The article "Optimal Allocation of Vaccine and Antiviral Drugs for Influenza Containment over Delayed Multiscale Epidemic Model considering Time-Dependent Transmission Rate" was published in 2021. Journal: Comput Math Methods Med.

# Optimal Allocation of Vaccine and Antiviral Drugs for Influenza Containment over Delayed Multiscale Epidemic Model considering Time-Dependent Transmission Rate

**DOI:** 10.1155/2021/4348910

**Published:** 2021-10-18

**Authors:** Zohreh Abbasi, Iman Zamani, Amir Hossein Amiri Mehra, Asier Ibeas, Mohsen Shafieirad

**Affiliations:** ^1^Department of Electrical and Computer Engineering, University of Kashan, Iran; ^2^Electrical and Electronic Engineering Department, Shahed University, Tehran, Iran; ^3^Departament de Telecomunicació i Enginyeria de Sistemes, Escolad'Enginyeria, Universitat Autònoma de Barcelona, Barcelona, Spain; ^4^Universidad de Bogotá Jorge Tadeo Lozano, Bogotá D.C., Colombia

## Abstract

In this study, two types of epidemiological models called “within host” and “between hosts” have been studied. The within-host model represents the innate immune response, and the between-hosts model signifies the SEIR (susceptible, exposed, infected, and recovered) epidemic model. The major contribution of this paper is to break the chain of infectious disease transmission by reducing the number of susceptible and infected people via transferring them to the recovered people group with vaccination and antiviral treatment, respectively. Both transfers are considered with time delay. In the first step, optimal control theory is applied to calculate the optimal final time to control the disease within a host's body with a cost function. To this end, the vaccination that represents the effort that converts healthy cells into resistant-to-infection cells in the susceptible individual's body is used as the first control input to vaccinate the susceptible individual against the disease. Moreover, the next control input (antiviral treatment) is applied to eradicate the concentrations of the virus and convert healthy cells into resistant-to-infection cells simultaneously in the infected person's body to treat the infected individual. The calculated optimal time in the first step is considered as the delay of vaccination and antiviral treatment in the SEIR dynamic model. Using Pontryagin's maximum principle in the second step, an optimal control strategy is also applied to an SEIR mathematical model with a nonlinear transmission rate and time delay, which is computed as optimal time in the first step. Numerical results are consistent with the analytical ones and corroborate our theoretical results.

## 1. Introduction

Seasonal and pandemic influenza A virus (IAV) infection causes severe morbidity and mortality worldwide [1]. There are many drugs to treat influenza, but the immune system is naturally the first defensive line against the disease. Therefore, it is essential to understand the mechanisms that trigger the immune system response and how this response affects the overall spread of the disease. The innate immune response plays an important role in the control and clearance of pathogens following viral infection inside an individual's body. However, in the majority of virus-infected individuals, the innate immune response is insufficient because viruses use different evasion strategies to escape the immune response. Innate immunity plays a critical role in the control of viral infection because most infectious pathogens are eliminated through innate immune response without necessarily requiring the activation of adaptive immunity [2].

The article "Optimal Allocation of Vaccine and Antiviral Drugs for Influenza Containment over Delayed Multiscale Epidemic Model considering Time-Dependent Transmission Rate" was published in 2021. Journal: Comput Math Methods Med.

Since innate immunity is an important part of the body for dealing with viral infections, some methods have been determined to model different aspects of the human immune system. Differential equation models are the most popular methods to simulate critical diseases' immunological and epidemiological dynamics [3]. In addition, the use of mathematical modeling of the innate immune response interpreting experimental results has made a significant contribution to this field. Many mathematical models of the immune response to IAV infection have been introduced that considered both different aspects of the immune system and different detail levels. The first mathematical model to illustrate the within-host dynamic of IAV in infected mice was developed in 1976 by Larson et al. [4]. The proposed compartmental model includes seven compartments with five associated rate parameters. Also, the virus population dynamic was introduced in mathematical terms. Another model introduced by Bocharov and Romanyukha [5] studied immune responses to viral infections in human infections, such as the influenza A virus, and considered 12 immune populations. Also, Baccam et al. [6] described the viral kinetics of influenza A during infection in the human body, including target cell and the innate interferon response with delayed virus production through infected cells. However, as opposed to previous papers, which did not consider a complete model of the innate immune system, we used a more comprehensive one adapted from [7].

However, the disease's impact within the community and the relationship between people in society also need to be examined. Mathematical models are instrumental in explaining and quantifying epidemic dynamics. Hence, various mathematical models have been proposed in the following for between-hosts epidemic models to provide a general overview of strategies to be employed in the period of influenza virus infection. Kermack and McKendrick created one of the simplest types to explain epidemic dynamics that is called SIR (susceptible, infected, and recovered individuals, respectively). The proposed model was described in three papers in 1927 [8], 1932 [9], and 1933 [10]. Moreover, in [11], another type of epidemic model (SIS) is considered with a nonlinear incidence rate and time delay. In addition, four different control strategies are investigated and compared, including optimal control to decrease the density of infected individuals, increase that of susceptible ones, and reduce relevant costs. Besides these, in [12], a model of the relationship between two types of systems is formulated and analyzed. The first dynamic is the within-host model dynamic and focuses on cellular interactions. The second is the between-hosts model dynamic that focuses on transmission and infection statuses that are governed by the susceptible-exposed-infected-recovered (SEIR) model. Likewise, in this study, motivated by the previous paper, a combined model with different relationships is presented that will be discussed in detail in the following sections. The authors in [13] have used the sliding mode control on the SEIAR dynamic to overcome the uncertainty of parameters. However, they have not considered the optimal time to eradicate the infection in society, and they only refer to the between-hosts dynamic. For this reason, since time is one of the priorities in order to control disease, we use an optimal control strategy to get the optimal time to cure the infected person and recover the susceptible person.

The article "Optimal Allocation of Vaccine and Antiviral Drugs for Influenza Containment over Delayed Multiscale Epidemic Model considering Time-Dependent Transmission Rate" was published in 2021. Journal: Comput Math Methods Med.

Optimal control is a mathematical method derived from the calculus of variations. There are different methods for computing the optimal control for mathematical models [14]. Pontryagin's maximum principle, first formulated in 1956 by L. S. Pontryagin [15], is to calculate the optimal control for an ordinary differential equation model system with a given constraint. In [16], an optimal control method is applied to a generic model of a pathogenic attack on the innate immune system. The minimization of a quadratic cost function is generated by numerical optimization. Terminal optimal time control is also investigated. For further studies, the readers are referred to [2], and the references therein introduce an optimal control model based on an ordinary differential equation system. Some studies have investigated the optimal control of SIR and SEIR models, but we mention just some of them in the following. The authors in [17] used an optimal control approach to an SIR epidemic model with a time delay to minimize the spread of infected individuals and maximize the number of susceptible and recovered individuals. Likewise, in [18, 19], optimal control is considered to minimize the level of infection at the terminal time for an SIR and SEIR model, respectively, where the incidence rate is an unspecified nonlinear function, while their models only consider one aspect of the impact of the disease that affects the community and the relationship between susceptible, infected, and recovered people. They do not take into account the effects of the disease inside the body, and the relationship between cells is not considered.

The article "Optimal Allocation of Vaccine and Antiviral Drugs for Influenza Containment over Delayed Multiscale Epidemic Model considering Time-Dependent Transmission Rate" was published in 2021. Journal: Comput Math Methods Med.

Epidemic mathematical models can be used for several epidemic diseases like COVID-19 by modifying the parameter and adding or eliminating some states. In this regard, the authors in [20] considered a SEIAR epidemic model for the COVID-19 pandemic. Also, some new SIR-type models are introduced in [21–24]. The authors in [21] have considered “isolated,” “vaccinated,” and “quarantined” people groups due to several different conditions (after and before vaccine development). Moreover, “hospitalized” and “ICU-admitted” people groups are introduced in [22] to express the spread of coronavirus between the healthcare workers. Also, in [23], a new epidemic model (called SIDARTHE) is studied that considers the distinction between diagnosed and nondiagnosed infected individuals with and without symptoms detected acutely symptomatic infected ones. Besides, the discrete-time SEIR epidemic models can be used in such studies instead of continuous ones [25, 26], to name a few. To further study about optimal control with time delay, readers refer to [27–31] and references therein.

Optimal control theory can be used to control other diseases like HIV [32] and especially COVID-19. In this regard, the authors in [33] used optimal control theory based on the SQEIAR epidemic model (Susceptible, Quarantined, Exposed, Infected, Asymptomatic, and Recovered) for the eradication of infection considering quarantine and treatment policies in China and Spain for different types of disease (COVID-19, Ebola, and influenza). Also, according to travel between cities that cause an increase in the outbreak, the authors in [33] investigated the impact of travel or immigration and impulsive change of population. These changes lead to generate impulsive epidemic models and impulsive control strategies [34]. Also, the authors in [35] have considered an optimal control strategy in the age-structured SEIRQ model for the COVID-19 epidemic in Brazil, where the quarantine entrance parameters are the control efforts of the system. In the same way, to explore the dynamic of the COVID-19 pandemic in Pakistan, the necessary optimality conditions are introduced in [36] using the optimal control theory in a mathematical model. Some optimal control strategies with application to COVID-19 are also introduced in [37], for further study.

The article "Optimal Allocation of Vaccine and Antiviral Drugs for Influenza Containment over Delayed Multiscale Epidemic Model considering Time-Dependent Transmission Rate" was published in 2021. Journal: Comput Math Methods Med.

This paper investigates the correlation between two modeling aspects: the effect of the disease on society and inside the individual's body, which is an important issue. The community includes four groups (SEIR), all of which relate to each other in a community. All communications occur only in the community and among individuals. In contrast, there are some interactions among the cells inside an individual's body. Recovering the susceptible by vaccination takes time that is considered as delay caused by the length of converting the healthy cells into resistant-to-infectious cells. Also, the infected people need to be treated with antiviral treatment to recover, which is also considered as a delay (the length of time to kill the infected and partially infected cells and viruses and convert the healthy cells into resistant-to-infection cells simultaneously).

The goal of the present paper will be presented clearly and thoroughly regarding the reviewed papers. This paper introduces a multiscale model in which both innate immune responses (within-host model) and the SEIR dynamic (between-hosts model) are used simultaneously to define a single system. A multiscale-type model has already been presented in [12], with the difference that the proposed model in the present study is more comprehensive and concisely describes the relationships between the virus, cells, and the immune system. The model is also more realistic and closer to the real world. Moreover, a nonlinear sinusoidal transmission rate (contact rate) is considered, which varies in time according to changes in contacts between people throughout day and night. In this study, the optimal control is used to eradicate the infection at the optimal time in the community. As discussed in Introduction, different papers have been published on the subject of optimal control. However, to the best of the authors' knowledge, an optimal control approach that simultaneously tackles both types of dynamics (within-host and between-hosts) for epidemic models has never been considered in the literature before.

1This paper is organized as follows.  Section 2 describes the preliminaries. After that, we propose an innate immune response dynamic in Section 3. The optimal control of innate immune response is introduced in Section 4, followed by the SEIR dynamic model with delay and nonlinear transmission rate in Section 5. In Section 6, we apply optimal control of the SEIR epidemic model. The results of simulations of different cases and sensitivity analysis are presented in Section 7. Finally, Section 8 summarizes the conclusions.

The article "Optimal Allocation of Vaccine and Antiviral Drugs for Influenza Containment over Delayed Multiscale Epidemic Model considering Time-Dependent Transmission Rate" was published in 2021. Journal: Comput Math Methods Med.

## 2. Preliminaries

In this section, we first look at the relationship between the two models considered in this paper. According to Figures 1 and 2, our multiscale model considers two scales: the first is the interaction of the virus and innate immune response within a host (inside the body), and the second is the contact between susceptible, exposed, infected, and recovered individuals in society. The dynamic of the innate immune response and relationship between cells and other components are now described in detail. The within-host model dynamic is the innate immune response to the influenza virus using a mathematical model. This model is based on interferon-induced resistance to infection of respiratory epithelial cells and the clearance of infected cells by natural killers with seven state variables (the numbers of healthy (*U*_*H*_), partially infected (*U*_*E*_), infected (*U*_*I*_), and resistant-to-infection cells (*U*_*R*_) and IFN-I molecules ([IFN]), natural killer cells (*K*), and virus particles (*V*)). Also, a nonlinear SEIR epidemiological model for influenza is given where the nonnegative state variables *S*(*t*), *E*(*t*), *I*(*t*), and *R*(*t*) are the susceptible, exposed, infected (symptomatic), and recovered compartments, respectively. Here, *S*(*t*) represents the number of people that are susceptible but not infected with influenza, *E*(*t*) denotes the number of people exposed to influenza (infected but not yet infectious), *I*(*t*) denotes the population of infected humans with infectious influenza symptoms, *R*(*t*) is the number of recovered people from influenza, and *N* is the total population size. The relationship between the two epidemic models is shown in Figures 1 and 2. The dynamics of the innate immune response and SEIR epidemiological model is described further in the following sections.

The general strategy for this study is described by the following Algorithm 1.

## 3. The Innate Immune Response Dynamic Model

In this section, we consider innate immune system dynamics for dealing with the influenza virus, which is derived from [7]. There are seven components to the dynamic states, and the following equations govern the dynamics. For brevity, we suppress the notation “(*t*)” for variables at the current time.

(1) $$\begin{array}{c} {\dot{U}}_{H}=S_{H}-k_{I}U_{H}V-k_{R}U_{H}\left[IFN\right]-\delta_{H}U_{H}, \end{array}$$

(2) $$\begin{array}{c} {\dot{U}}_{E}=k_{I}U_{H}V-k_{E}U_{E}-q_{K}U_{E}K, \end{array}$$

(3) $$\begin{array}{c} {\dot{U}}_{I}=k_{E}U_{E}-\delta_{I}U_{I}-q_{K}U_{I}K, \end{array}$$

(4) $$\begin{array}{c} {\dot{U}}_{R}=k_{R}U_{H}\left[IFN\right]-\delta_{R}U_{R}, \end{array}$$

(5) $$\begin{array}{c} \dot{V}=\rho_{V}U_{I}-\delta_{V}V, \end{array}$$

(6) $$\begin{array}{c} \dot{\left[IFN\right]}=a_{I}U_{I}-\delta_{IFN}\left[IFN\right], \end{array}$$

(7) $$\begin{array}{c} \dot{K}=S_{K}+\Phi_{K}U_{I}-\delta_{K}K, \end{array}$$

where *U*_*H*_ is the number of healthy cells that increase with cell growth rate *S*_*H*_. These cells become partially infected cells (*U*_*E*_) via the virus particles (*V*) with rate *k*_*I*_. They also convert to resistant-to-infection cells (*U*_*R*_) by the rate *k*_*R*_ with IFN-I molecules ([IFN]) that increase by the rate of *a*_*I*_. Partially infected cells are in the eclipse phase. This means that they cannot spread the virus in the body and they infect the other healthy cells by the term *k*_*E*_. When the partially infected cells pass through the eclipse phase, they will become infected cells (*U*_*I*_) and can spread the virus and cause other healthy cells to become infected. Partially infected (*U*_*E*_) and infected cells (*U*_*I*_) are destroyed by natural killers (*K*) at a rate of *q*_*K*_. Once the cells are infected (*U*_*I*_), they broadcast thousands of similar cells a day, which is denoted by the parameter *ρ*_*V*_. The natural death rates of healthy, infected, infection-resistant cells, and IFN-I molecules are denoted by *δ*_*H*_, *δ*_*I*_, *δ*_*R*_, and *δ*_IFN_, respectively, and the clear rate of virus particles (*V*) is *δ*_*V*_. The number of NKs (natural killers) increases with a constant cell growth rate *S*_*K*_. In the same way, NKs die at the rate of *δ*_*K*_. After inflammatory stimulation caused by infected cells, natural killers are recruited from the blood indicated by *Φ*_*K*_*U*_*I*_.  Figure 3 shows a schematic diagram of the innate immune system response to the influenza virus, which shows the cells' relation very well.

The article "Optimal Allocation of Vaccine and Antiviral Drugs for Influenza Containment over Delayed Multiscale Epidemic Model considering Time-Dependent Transmission Rate" was published in 2021. Journal: Comput Math Methods Med.

After introducing the model, we now introduce the controller and investigate how to influence the vaccine and antiviral treatment on the cells. As mentioned earlier, the vaccination is used to make healthy cells resistant to infection in a susceptible person's body and by using the antiviral treatment, the virus particles, infected, and partially infected cells are removed inside the infected body as discussed in detail in the next section.

### 3.1. Equilibrium Points and the Basic Reproduction Number

To determine the disease spread and the number of secondary infections, an infected individual would produce in his/her infectious period the most important threshold criterion named “the basic reproduction number” (*R*_0_) can be calculated as the follows.

According to the definition of *R*_0_ = *ρ*(*FV*^−1^), where

(8) $$\begin{array}{c} F=\left[\begin{array}{ccc} 0 & 0 & k_{I}\frac{S_{H}}{\delta_{H}}\\ 0 & 0 & 0\\ 0 & 0 & 0 \end{array}\right],\\ V=\left[\begin{array}{ccc} k_{E}+q_{K}\frac{S_{K}}{\delta_{K}} & 0 & 0\\ -k_{E} & \delta_{I}+q_{K}\frac{S_{K}}{\delta_{K}} & 0\\ 0 & -\rho_{V} & \delta_{V} \end{array}\right], \end{array}$$

*R*_0_ is calculated as *R*_0_ = *δ*_*H*_*S*_*H*_*k*_*I*_*k*_*E*_*ρ*_*V*_*δ*_*K*_^2^/(*δ*_*V*_(*k*_*E*_*δ*_*K*_ + *q*_*K*_*S*_*K*_)(*δ*_*I*_*δ*_*K*_ + *q*_*K*_*S*_*K*_)).

The disease-free equilibrium point (DFE) is calculated by equating Equations (1)–(7) to zero and solving for *U*_*E*_^∗^ = *U*_*I*_^∗^ = *V*^∗^ = [IFN]^∗^ = 0 as (*S*_*H*_/*δ*_*H*_, 0, 0, 0, 0, 0, 0, *S*_*K*_/*δ*_*K*_). To find the endemic equilibrium point (EE), Equations (1)–(7) are equated to zero, *U*_*H*_ = *S*_*H*_/(*k*_*I*_*V* + *k*_*R*_[IFN] + *δ*_*H*_), *U*_*E*_ = *k*_*I*_*U*_*H*_*V*/(*k*_*E*_ + *q*_*K*_*K*), *U*_*I*_ = *k*_*E*_*U*_*E*_/(*δ*_*I*_ + *q*_*K*_*K*), *U*_*R*_ = (*k*_*R*_*U*_*H*_[IFN])/*δ*_*R*_, *V* = *ρ*_*V*_*U*_*I*_/*δ*_*V*_, and [IFN] = *a*_*I*_*U*_*I*_/*δ*_IFN_. Therefore, by replacing the states, the following equations can be calculated: ${\bar{U}}_{H}=S_{H}/\left(a_{1}{\bar{U}}_{I}+\delta_{H}\right)$, ${\bar{U}}_{E}=a_{2}/\left(a_{3}\delta_{H}+a_{5}{\bar{U}}_{I}-a_{1}a_{4}{\bar{U}}_{I}^{2}\right){\bar{U}}_{I}$, ${\bar{U}}_{R}=k_{R}S_{H}\delta_{V}a_{I}/\left(a_{7}{\bar{U}}_{I}-\delta_{H}\delta_{V}\delta_{R}\delta_{\text{IFN}}\right){\bar{U}}_{I}$, $\bar{V}=\left(\rho_{V}/\delta_{V}\right){\bar{U}}_{I}$, $\left[\bar{\text{IFN}}\right]=\left(a_{I}/\delta_{\text{IFN}}\right){\bar{U}}_{I}$, $\bar{K}=\left(S_{K}+\Phi_{K}{\bar{U}}_{I}\right)/\delta_{K}$, and $\alpha_{1}{\bar{U}}_{I}^{4}+\alpha_{2}{\bar{U}}_{I}^{3}+\alpha_{3}{\bar{U}}_{I}^{2}+\alpha_{4}{\bar{U}}_{I}=0$. The last equation has four solutions that one of them is DFE and can be achieved by ${\bar{U}}_{I}=0$. The other three solutions are obtained using the parameter values in Table 1, one of which is  1.84 × 10^5^, and the other two solutions are negative and unacceptable, because the number of cells is a positive value. Therefore, the other equilibrium points are given as $\text{EE}=\left({\bar{U}}_{H},{\bar{U}}_{E},{\bar{U}}_{I},{\bar{U}}_{R},\bar{V},\left[\bar{\text{IFN}}\right],\bar{K}\right)=\left(S_{H}/\left(a_{1}{\bar{U}}_{I}+\delta_{H}\right),a_{2}/\left(a_{3}\delta_{H}+a_{5}{\bar{U}}_{I}-a_{1}a_{4}{\bar{U}}_{I}^{2}\right){\bar{U}}_{I},{\bar{U}}_{I},k_{R}S_{H}\delta_{V}a_{I}/\left(a_{7}{\bar{U}}_{I}-\delta_{H}\delta_{V}\delta_{R}\delta_{\text{IFN}}\right){\bar{U}}_{I},\left(\rho_{V}/\delta_{V}\right){\bar{U}}_{I},\left(a_{I}/\delta_{\text{IFN}}\right){\bar{U}}_{I},\left(S_{K}+\Phi_{K}{\bar{U}}_{I}\right)/\delta_{K}\right)$, in which, *α*_1_ = *q*_*K*_^2^*Φ*_*K*_^2^/*δ*_*K*_^2^*δ*_IFN_(*δ*_IFN_*k*_*I*_*ρ*_*V*_ + *k*_*R*_*δ*_*I*_*δ*_*V*_), *α*_2_ = *q*_*K*_*Φ*_*K*_/*δ*_*K*_^2^*δ*_IFN_(2*δ*_IFN_*k*_*I*_*ρ*_*V*_*q*_*K*_*S*_*K*_ + *δ*_*K*_*δ*_IFN_*k*_*I*_*ρ*_*V*_(*k*_*E*_ + *δ*_*I*_) + 2*q*_*K*_*k*_*R*_*S*_*K*_*δ*_*V*_*a*_*I*_ + *k*_*R*_*δ*_*V*_*δ*_*K*_*a*_*I*_(*k*_*E*_ + *δ*_*I*_) + *δ*_*H*_*δ*_*V*_*δ*_IFN_*q*_*K*_*Φ*_*K*_), *α*_3_ = 1/*δ*_*K*_^2^*δ*_IFN_(*k*_*I*_*ρ*_*V*_(*δ*_*K*_^2^*δ*_IFN_*k*_*E*_*δ*_*I*_ + *δ*_*K*_*δ*_IFN_*q*_*K*_*S*_*K*_(*k*_*E*_ + *δ*_*I*_) + *q*_*K*_^2^*δ*_IFN_*S*_*K*_^2^) + *k*_*R*_*a*_*I*_(*δ*_*K*_^2^*δ*_*V*_*k*_*E*_*δ*_*I*_ + *δ*_*K*_*δ*_*V*_*q*_*K*_*S*_*K*_(*k*_*E*_ + *δ*_*I*_) + *q*_*K*_^2^*δ*_*V*_*S*_*K*_^2^) + *δ*_*H*_*δ*_*V*_*q*_*K*_*Φ*_*K*_(2*δ*_IFN_*q*_*K*_*S*_*K*_ + *δ*_*K*_*δ*_IFN_(*k*_*E*_ + *δ*_*I*_))), and *α*_4_ = (1/*δ*_*K*_^2^)(*k*_*E*_*δ*_*I*_*δ*_*H*_*δ*_*V*_*δ*_*K*_^2^ + *δ*_*K*_*δ*_*H*_*δ*_*V*_*q*_*K*_*S*_*K*_(*k*_*E*_ + *δ*_*I*_) + *δ*_*H*_*q*_*K*_^2^*δ*_*V*_*S*_*K*_^2^ − *k*_*E*_*k*_*I*_*ρ*_*V*_*S*_*H*_).

The article "Optimal Allocation of Vaccine and Antiviral Drugs for Influenza Containment over Delayed Multiscale Epidemic Model considering Time-Dependent Transmission Rate" was published in 2021. Journal: Comput Math Methods Med.

Then, the Jacobian of Equations (1)–(7) is given by

(9) $$\begin{array}{c} J=\left[\begin{array}{ccccccc} -k_{I}V-k_{R}\left[IFN\right]-\delta_{H} & 0 & 0 & 0 & -k_{I}U_{H} & -k_{R}U_{H} & 0\\ k_{I}V & -k_{E}-q_{K}K & 0 & 0 & -k_{I}U_{H} & 0 & -q_{K}U_{E}\\ 0 & k_{E} & -\delta_{I}-q_{K}K & 0 & 0 & 0 & -q_{K}U_{I}\\ k_{R}\left[IFN\right] & 0 & 0 & -\delta_{R} & 0 & k_{R}U_{H} & 0\\ 0 & 0 & \rho_{V} & 0 & -\delta_{V} & 0 & 0\\ 0 & 0 & a_{I} & 0 & 0 & -\delta_{IFN} & 0\\ 0 & 0 & \Phi_{K} & 0 & 0 & 0 & -\delta_{K} \end{array}\right]. \end{array}$$

**Theorem 1 .**

The DFE is locally stable if *R*_0_ < 1 while it is unstable if *R*_0_ > 1.

**Proof**

By calculating the seventh-order characteristic equation of *J* about its DFE and according to the Routh-Hurwitz criterion, the following inequality must be satisfied:

(10) $$\begin{array}{c} \delta_{V}\left(k_{E}\delta_{K}+q_{K}S_{K}\right)\left(\delta_{I}\delta_{K}+q_{K}S_{K}\right)-\delta_{H}S_{H}k_{I}k_{E}\rho_{V}{\delta_{K}}^{2}>0. \end{array}$$

Therefore, it can be concluded that *R*_0_ < 1. For *R*_0_ > 1, there exists a positive eigenvalue for the characteristic equation and the equilibrium point is unstable.

**Theorem 2 .**

The EE is locally stable if *R*_0_ > 1 and unstable if *R*_0_ < 1.

**Proof**

In the same way and by calculating the characteristic equation of *J* about its EE and according to the negative eigenvalues obtained from Jacobian, the EE is stable if *R*_0_ > 1, otherwise it is unstable.

### 3.2. Sensitivity Analysis

In this subsection, the sensitivity of *R*_0_ is investigated. Therefore, to check the *R*_0_ sensitivity, *S*_*α*_^*R*_0_^ = (*∂R*_0_/*∂α*)(*α*/*R*_0_), we have

(11) $$\begin{array}{c} S_{\delta_{H}}^{R_{0}}=1,\\ S_{S_{H}}^{R_{0}}=1,\\ S_{k_{I}}^{R_{0}}=1,\\ S_{\rho_{V}}^{R_{0}}=1,\\ S_{k_{E}}^{R_{0}}=\frac{q_{K}S_{K}}{\left(k_{E}\delta_{K}+q_{K}S_{K}\right)},\\ S_{\delta_{K}}^{R_{0}}=\frac{q_{K}S_{K}\left(k_{E}\delta_{K}+\delta_{I}\delta_{K}+2S_{K}q_{K}\right)}{\left(k_{E}\delta_{K}+q_{K}S_{K}\right)\left(\delta_{K}\delta_{I}+q_{K}S_{K}\right)},\\ S_{\delta_{V}}^{R_{0}}=-\delta_{V}\left(k_{E}\delta_{K}+q_{K}S_{K}\right)\left(\delta_{I}\delta_{K}+q_{K}S_{K}\right),\\ S_{q_{K}}^{R_{0}}=\frac{-q_{K}\left(k_{E}\delta_{K}S_{K}\delta_{V}+S_{K}\delta_{I}\delta_{K}\delta_{V}+2\delta_{V}S_{K}^{2}q_{K}\right)}{\delta_{V}\left(k_{E}\delta_{K}+q_{K}S_{K}\right)\left(\delta_{I}\delta_{K}+q_{K}S_{K}\right)},\\ S_{S_{K}}^{R_{0}}=\frac{-S_{K}\left(k_{E}\delta_{K}q_{K}\delta_{V}+q_{K}\delta_{I}\delta_{K}\delta_{V}+2\delta_{V}S_{K}q_{K}^{2}\right)}{\delta_{V}\left(k_{E}\delta_{K}+q_{K}S_{K}\right)\left(\delta_{I}\delta_{K}+q_{K}S_{K}\right)}. \end{array}$$

It can be concluded that *R*_0_ is directly related to the change of parameters *δ*_*H*_, *S*_*H*_, *k*_*I*_, *ρ*_*V*_, *k*_*E*_, and *δ*_*K*_. That is, if the parameters *δ*_*H*_, *S*_*H*_, *k*_*I*_, and *ρ*_*V*_ increase by 10%, *R*_0_ also changes accordingly (10%) and is inversely related to the parameters *δ*_*V*_, *q*_*K*_, and *S*_*K*_.

The article "Optimal Allocation of Vaccine and Antiviral Drugs for Influenza Containment over Delayed Multiscale Epidemic Model considering Time-Dependent Transmission Rate" was published in 2021. Journal: Comput Math Methods Med.

### 3.3. Positivity Analysis

In this subsection, the positivity of solutions is investigated with Theorem 3.

**Theorem 3 .**

If *U*_*H*__0_ ≥ 0, *U*_*E*__0_ ≥ 0, *U*_*I*__0_ ≥ 0, *U*_*R*_0__ ≥ 0, *V*_0_ ≥ 0, [IFN]_0_ ≥ 0, and *K*_0_ ≥ 0, then solutions of the model are positive for all *t* ≥ 0.

**Proof**

According to the positivity of all the parameters of the model, Equation (4) can be written as ${\dot{U}}_{R}\left(t\right)\geq -\delta_{R}U_{R}\left(t\right)$. Multiplying *e*^∫_0_^*t*^*δ*_*R*_*dr*^ into two both side gives ${\dot{U}}_{R}\left(t\right)e^{\int_{0}^{t}\delta_{R}dr}+\delta_{R}U_{R}\left(t\right)e^{\int_{0}^{t}\delta_{R}dr}\geq 0$; then, (*d*/*dt*)(*e*^∫_0_^*t*^*δ*_*R*_*dr*^*U*_*R*_(*t*)) ≥ 0; integrating from 0 to *t* gives *U*_*R*_(*t*) ≥ *U*_*R*_(0)*e*^−∫_0_^*t*^*δ*_*R*_*dr*^ ≥ 0. Therefore *U*_*R*_(*t*) is positive (*U*_*R*_(*t*) ≥ 0). In the same way, the other states *V*(*t*), [IFN](*t*), and *K*(*t*) (Equations (5)–(7)) are also positive states and can be written as *V*(*t*) ≥ *V*(0)*e*^−∫_0_^*t*^*δ*_*V*_*dr*^ ≥ 0, [IFN](*t*) ≥ [IFN](0)*e*^−∫_0_^*t*^*δ*_IFN_*dr*^ ≥ 0, and  *K*(*t*) ≥ *K*(0)*e*^−∫_0_^*t*^*δ*_*K*_*dr*^ ≥ 0. According to the positivity of *U*_*R*_(*t*), *V*(*t*), [IFN](*t*) and *K*(*t*) and according to Equation (3), *U*_*I*_(*t*) ≥ *U*_*I*_(0)*e*^−∫_0_^*t*^(*δ*_*I*_ + *q*_*K*_*K*)*dr*^ ≥ 0; therefore, *U*_*I*_(*t*) ≥ 0. Similarly, *U*_*E*_(*t*) ≥ *U*_*E*_(0)*e*^−∫_0_^*t*^(*k*_*E*_ + *q*_*K*_*K*)*dr*^ ≥ 0 and *U*_*H*_(*t*) ≥ *U*_*H*_(0)*e*^−∫_0_^*t*^(−*k*_*I*_*V* − *k*_*R*_[IFN] − *δ*_*H*_)*dr*^ ≥ 0. Therefore, all solutions are positive.

The article "Optimal Allocation of Vaccine and Antiviral Drugs for Influenza Containment over Delayed Multiscale Epidemic Model considering Time-Dependent Transmission Rate" was published in 2021. Journal: Comput Math Methods Med.

### 3.4. Existence of Solutions

In this subsection, the existence of solutions is investigated with Theorem 4.

**Theorem 4 .**

The proposed model with the initial conditions *U*_*H*_(0) ≥ 0, *U*_*E*_(0) ≥ 0, *U*_*I*_(0) ≥ 0, *U*_*R*_(0) ≥ 0, *V*(0) ≥ 0, [IFN](0) ≥ 0, *K*(0) ≥ 0, and *E*(0) ≥ 0 has a unique solution.

**Proof**

The model can be rewritten as

(12) $$\begin{array}{c} f\left(X\right)=AX+f_{1}\left(X\right) \end{array}$$

where $X={\left[U_{H}\left(t\right)\;U_{E}\left(t\right)\;U_{I}\left(t\right)\;\begin{array}{ccc} U_{R}\left(t\right) & V\left(t\right) & \left[\text{IFN}\right]\left(t\right)\;K\left(t\right) \end{array}\right]}^{T}$ and *𝒜* = diag $\left[\begin{array}{ccc} -\delta_{H}, & -k_{E}, & -\delta_{I} \end{array},\begin{array}{ccc} -\delta_{R}, & -\delta_{V}, & -\delta_{\text{IFN}} \end{array},-\delta_{K}\right]$and $f_{1}\left(X\right)={\left[\begin{array}{ccc} S_{H}-k_{I}U_{H}V-k_{R}U_{H}\left[\text{IFN}\right] & k_{I}U_{H}V-q_{K}U_{E}K & k_{E}U_{E}-q_{K}U_{I}K \end{array}\;\begin{array}{ccc} k_{R}U_{H}\left[\text{IFN}\right] & \rho_{V}U_{I} & a_{I}U_{I}\;S_{K}+\Phi_{K}U_{I}\; \end{array}\right]}^{T}$.

The function *f*_1_(*X*) satisfies

(13) $$\begin{array}{c} \left|f_{1}\left(X_{1}\right)-f_{1}\left(X_{2}\right)\right|=\left|k_{I}\left({U_{H}}_{2}V_{2}-{U_{H}}_{1}V_{1}\right)\right|+\left|k_{I}\left({U_{H}}_{1}V_{1}-{U_{H}}_{2}V_{2}\right)\right|+\left|k_{R}\left({U_{H}}_{2}{\left[\text{IFN}\right]}_{2}-{U_{H}}_{1}{\left[\text{IFN}\right]}_{1}\right)\right|+\left|q_{K}\left({U_{E}}_{2}K_{2}-{U_{E}}_{1}K_{1}\right)\right|+\left|k_{E}\left(-{U_{E}}_{2}+{U_{E}}_{1}\right)\right|+\left|q_{K}\left({U_{I}}_{2}K_{2}-{U_{I}}_{1}K_{1}\right)\right|+\left|k_{R}\left({U_{\text{H}}}_{1}{\left[\text{IFN}\right]}_{1}-{U_{H}}_{2}{\left[\text{IFN}\right]}_{2}\right)\right|+\left|\left(\rho_{V}+a_{I}+\Phi_{K}\right)\left({U_{I}}_{1}-{U_{I}}_{2}\right)\right| \end{array}$$

Assumed that all parameters have the maximum value *ℳ* which is a bounded value:

(14) $$\begin{array}{c} \left|f_{1}\left(X_{1}\right)-f_{1}\left(X_{2}\right)\right|\leq \left|M\left({U_{H}}_{1}V_{1}-{U_{H}}_{2}V_{2}\right)\right|+\left|M\left({U_{H}}_{1}{\left[\text{IFN}\right]}_{1}-{U_{H}}_{2}{\left[\text{IFN}\right]}_{2}\right)\right|+\left|M\left({U_{E}}_{1}K_{1}-{U_{E}}_{2}K_{2}\right)\right|+\left|M\left({U_{I}}_{1}K_{1}-{U_{I}}_{2}K_{2}\right)\right|+\left|M\left({U_{E}}_{1}-{U_{E}}_{2}\right)\right|+\left|M\left({U_{I}}_{1}-{U_{I}}_{2}\right)\right|. \end{array}$$

Replacing (*U*_*H*__1_*V*_1_ − *U*_*H*__2_*V*_2_) by (*U*_*H*__1_*V*_1_ − *U*_*H*__2_*V*_1_ + *U*_*H*__2_*V*_1_ − *U*_*H*__2_*V*_2_) and similarly for others,

(15) $$\begin{array}{c} \left|f_{1}\left(X_{1}\right)-f_{1}\left(X_{2}\right)\right|\leq \left|M\left({U_{H}}_{1}V_{1}-{U_{H}}_{2}V_{1}+{U_{H}}_{2}V_{1}-{U_{H}}_{2}V_{2}\right)\right|+\left|M\left({U_{H}}_{1}{\left[\text{IFN}\right]}_{1}-{U_{H}}_{2}{\left[\text{IFN}\right]}_{1}+{U_{H}}_{2}{\left[\text{IFN}\right]}_{1}-{U_{H}}_{2}{\left[\text{IFN}\right]}_{2}\right)\right|+\left|M\left({U_{E}}_{1}K_{1}-{U_{E}}_{2}K_{1}+{U_{E}}_{2}K_{1}-{U_{E}}_{2}K_{2}\right)\right|+\left|M\left({U_{I}}_{1}K_{1}-{U_{I}}_{2}K_{1}+{U_{I}}_{2}K_{1}-{U_{I}}_{2}K_{2}\right)\right|+\left|M\left({U_{E}}_{1}-{U_{E}}_{2}\right)\right|+\left|M\left({U_{I}}_{1}-{U_{I}}_{2}\right)\right| \end{array}$$

Therefore,

(16) $$\begin{array}{c} \left|f_{1}\left(X_{1}\right)-f_{1}\left(X_{2}\right)\right|\leq \left|MV_{1}\left({U_{H}}_{1}-{U_{H}}_{2}\right)+M{U_{H}}_{2}\left(V_{1}-V_{2}\right)\right|+\left|M{\left[\text{IFN}\right]}_{1}\left({U_{H}}_{1}-{U_{H}}_{2}\right)+{{MU}_{H}}_{2}\left({\left[\text{IFN}\right]}_{1}-{\left[\text{IFN}\right]}_{2}\right)\right|+\left|MK_{1}\left({U_{E}}_{1}-{U_{E}}_{2}\right)+M{U_{E}}_{2}\left(K_{1}-K_{2}\right)\right|+\left|MK_{1}\left({U_{I}}_{1}-{U_{I}}_{2}\right)+M{U_{I}}_{2}\left(K_{1}-K_{2}\right)\right|+\left|M\left({U_{E}}_{1}-{U_{E}}_{2}\right)\right|+\left|M\left({U_{I}}_{1}-{U_{I}}_{2}\right)\right|. \end{array}$$

The maximum value of states is equal to *ℛ* (bounded value); therefore,

(17) $$\begin{array}{c} \left|f_{1}\left(X_{1}\right)-f_{1}\left(X_{2}\right)\right|\leq 2RM\left|{U_{H}}_{1}-{U_{H}}_{2}\right|+RM\left|V_{1}-V_{2}\right|+RM\left|{\left[\text{IFN}\right]}_{1}-{\left[\text{IFN}\right]}_{2}\right|+2RM\left|{U_{I}}_{1}-{U_{I}}_{2}\right|+2RM\left|K_{1}-K_{2}\right|+2RM\left|{U_{E}}_{1}-{U_{E}}_{2}\right|\leq 2RM\left|X_{1}-X_{2}\right|. \end{array}$$

It can be concluded that ‖*f*_1_(*X*_1_) − *f*_1_(*X*_2_)‖ ≤ 2*ℛℳ*‖*X*_1_ − *X*_2_‖. Therefore, ‖*f*(*X*_1_) − *f*(*X*_2_)‖ ≤ *L*‖*X*_1_ − *X*_2_‖, where *L* = max(2*ℛℳ*, ‖*𝒜*‖). Thus, *f* is uniformly Lipschitz continuous, and the solutions exist.

The article "Optimal Allocation of Vaccine and Antiviral Drugs for Influenza Containment over Delayed Multiscale Epidemic Model considering Time-Dependent Transmission Rate" was published in 2021. Journal: Comput Math Methods Med.

## 4. Optimal Control of Within-Host Epidemic Model

Optimal control techniques are used to improve optimal strategies to control numerous kinds of diseases. The flexibility and relative simplicity of optimal control techniques can lead to the development of the optimal strategies to control the monitoring and treating of various kinds of diseases [14]. Therefore, the optimal control theory is applied to the innate immune dynamic in this part of the paper. In the first subsection, the optimal control is used to vaccinate susceptible people and cure infected people.

### 4.1. Vaccination Strategy

In this subsection, the optimal control is applied to the innate immune response to convert healthy cells to resistant-to-infection cells. The vaccine works with the innate immune to develop protection (immunity) to the disease. This subsection is aimed at minimizing the number of healthy cells (*U*_*H*_) by converting them to resistant-to-infection cells (*U*_*R*_) with the control input (vaccination) at a rate of *ν* in the optimal time. It is obvious that injecting a vaccine into the susceptible person's bodies takes time to vaccinate them (recovered) against the disease. Unlike [13, 19], in the current paper, this time is considered as a delay in moving susceptible people to the recovered people group in the society, which is investigated in Section 5 in detail. As long as the healthy cells have not become resistant-to-infection cells in the susceptible body, the person has not been vaccinated against the disease, and there is still a risk of infection. The above description is given by the following model:

(18) $$\begin{array}{c} {\dot{U}}_{H}=S_{H}-k_{I}U_{H}V-k_{R}U_{H}\left[\text{IFN}\right]-\delta_{H}U_{H}-\nu U_{H}, \end{array}$$

(19) $$\begin{array}{c} {\dot{U}}_{E}=k_{I}U_{H}V-k_{E}U_{E}-q_{K}U_{E}K, \end{array}$$

(20) $$\begin{array}{c} {\dot{U}}_{I}=k_{E}U_{E}-\delta_{I}U_{I}-q_{K}U_{I}K, \end{array}$$

(21) $$\begin{array}{c} {\dot{U}}_{R}=k_{R}U_{H}\left[\text{IFN}\right]-\delta_{R}U_{R}+\nu U_{H}, \end{array}$$

(22) $$\begin{array}{c} \dot{V}=\rho_{V}U_{I}-\delta_{V}V, \end{array}$$

(23) $$\begin{array}{c} \dot{\left[\text{IFN}\right]}=a_{I}U_{I}-\delta_{\text{IFN}}\left[\text{IFN}\right], \end{array}$$

(24) $$\begin{array}{c} \dot{K}=S_{K}+\Phi_{K}U_{I}-\delta_{K}K. \end{array}$$

Figure 3 shows the diagram of the within-host dynamic model with vaccination. The susceptible individual's body does not have the virus, infected, or partially infected cells. Therefore, the goal is to convert healthy cells into resistant-to-infection cells using the vaccination strategy in the optimal time.

Therefore, the optimal control problem is to minimize the cost (objective) function applied to Equations (18)–(24) given by

(25) $$\begin{array}{c} J\left(\nu ,t_{f}\right)=\int_{0}^{t_{f}}\left[A_{1}U_{H}-A_{2}U_{R}+\frac{A_{3}}{2}\nu^{2}\right]dt+\emptyset \left(t_{f}\right), \end{array}$$

in which a free terminal time is investigated, which gives a minimum duration of a vaccination. *t*_*f*_ represent the duration of the vaccination. ∅ is a positive increasing function such that $\underset{t⟶\infty }{\lim}\emptyset \left(t\right)=+\infty$. In other words, the vaccination strategy is applied using the optimal control (*ν*^∗^) in optimal time (*t*_*f*_^∗^) such that

(26) $$\begin{array}{c} J\left(\nu^{*},{t_{f}}^{*}\right)=\min\left\{J\left(\nu ,t_{f}\right)\;|\;\nu \in U_{1},t_{f}\in {\mathbb{R}}^{+}\right\}, \end{array}$$

where *ν* is control and *U*_1_ is the set of admissible controls defined by

(27) $$\begin{array}{c} U_{1}=\left\{U_{1}\text{ is measurable},\;0\leq \nu \leq \nu_{\max}=1,t\in \left[0,t_{f}\right]\right\}. \end{array}$$

The necessary conditions for optimality are expressed by

(28) $$\begin{array}{c} {\left[\nabla_{X_{f}}^{\emptyset }-p\left(t_{f}\right)\right]}^{T}\delta X_{f}+\left[H\left(X\left(t_{f}\right),u\left(t_{f}\right),p\left(t_{f}\right),t_{f}\right)+\frac{\partial \emptyset }{\partial t_{f}}\right]{\delta t}_{f}=0, \end{array}$$

where *X*(*t*_*f*_) or *X*_*f*_ is vector of constant values (the final value of all states is known). The gradient (∇_*X*_*f*__^∅^) is the derivative of ∅(*t*_*f*_). *t*_*f*_ is unknown but *X*(*t*_*f*_) is defined; therefore, *δX*_*f*_ = 0. Also, a stationarity condition on the control is as follows:

(29) $$\begin{array}{c} \nabla_{\nu }^{H}=0, \end{array}$$

which are expressed using the Hamiltonian of the system. The Hamiltonian for the control problem is defined as follows:

(30) $$\begin{array}{c} H=g+p^{T}f, \end{array}$$

where $f=\dot{x}={\left[{\dot{U}}_{H},{\dot{U}}_{E},{\dot{U}}_{I},{\dot{U}}_{R},\dot{V},\dot{\left[\text{IFN}\right]},\dot{K}\right]}^{T}$ and *g* = [*A*_1_*U*_*H*_ − *A*_2_*U*_*R*_ + (*A*_3_/2)*ν*^2^].

The article "Optimal Allocation of Vaccine and Antiviral Drugs for Influenza Containment over Delayed Multiscale Epidemic Model considering Time-Dependent Transmission Rate" was published in 2021. Journal: Comput Math Methods Med.

Therefore,

(31) $$\begin{array}{c} H=A_{1}U_{H}-A_{2}U_{R}+\frac{A_{3}}{2}\nu^{2}+p_{1}{\dot{U}}_{H}+p_{2}{\dot{U}}_{E}+p_{3}{\dot{U}}_{I}+p_{4}{\dot{U}}_{R}+p_{5}\dot{V}+p_{6}\dot{\left[\text{IFN}\right]}+p_{7}\dot{K,} \end{array}$$

and *p*_1_, *p*_2_, *p*_3_, *p*_4_, *p*_5_, *p*_6_, and *p*_7_ are the adjoint functions to be determined suitably. Then, the necessary conditions are computed as follows:

(32) $$\begin{array}{c} \dot{x}=\frac{\partial H}{\partial p}={\left[{\dot{U}}_{H},{\dot{U}}_{E},{\dot{U}}_{I},{\dot{U}}_{R},\dot{V},\dot{\left[\text{IFN}\right]},\dot{K}\right]}^{T}. \end{array}$$

Then, the necessary conditions for optimality are computed, which are expressed by the mentioned Hamiltonian equations [38]. These equations include a linear, ordinary differential equation that are shown by

(33) $$\begin{array}{c} \dot{p}=-\frac{\partial H}{\partial x}={\left[-\frac{\partial H}{\partial U_{H}},-\frac{\partial H}{\partial U_{E}},-\frac{\partial H}{\partial U_{I}},-\frac{\partial H}{\partial U_{R}},-\frac{\partial H}{\partial V},-\frac{\partial H}{\partial \left[\text{IFN}\right]},-\frac{\partial H}{\partial K}\right]}^{T}. \end{array}$$

In order to derive the necessary conditions for this optimal control, the Pontryagin maximum principle [39] is applied to characterize the optimal control problem and the optimal final time, which is given as the following theorem.

The article "Optimal Allocation of Vaccine and Antiviral Drugs for Influenza Containment over Delayed Multiscale Epidemic Model considering Time-Dependent Transmission Rate" was published in 2021. Journal: Comput Math Methods Med.

**Theorem 5 .**

Given an optimal control *ν*^∗^, solutions *U*_*H*_^∗^, *U*_*E*_^∗^, *U*_*I*_^∗^, *U*_*R*_^∗^, *V*^∗^, [IFN]^∗^, and *K*^∗^ for the optimal control problem *J*(*ν*^∗^, *t*_*f*_^∗^) = min{*J*(*ν*, *t*_*f*_) | *ν* ∈ *U*_1_, *t*_*f*_ ∈ ℝ^+^}. Then, there are adjoint variables *p*_1_, *p*_2_, *p*_3_, *p*_4_, *p*_5_, *p*_6_, and *p*_7_ that satisfy

(34) $$\begin{array}{c} {\dot{p}}_{1}=-A_{1}+p_{1}\delta_{H}-k_{I}V\left[p_{2}-p_{1}\right]-\left[k_{R}\left[\text{IFN}\right]+\nu \right]\left[p_{4}-p_{1}\right], \end{array}$$

(35) $$\begin{array}{c} {\dot{p}}_{2}=p_{2}\left[k_{E}+q_{K}K\;\right]-p_{3}k_{E}, \end{array}$$

(36) $$\begin{array}{c} {\dot{p}}_{3}=p_{3}\left[\delta_{I}+q_{K}K\;\right]-p_{5}\rho_{V}-p_{6}a_{I}-p_{7}\Phi_{K}, \end{array}$$

(37) $$\begin{array}{c} {\dot{p}}_{4}=A_{2}+p_{4}\delta_{R}, \end{array}$$

(38) $$\begin{array}{c} {\dot{p}}_{5}=k_{I}U_{H}\left[p_{2}+p_{1}\right]+p_{5}\rho_{V}, \end{array}$$

(39) $$\begin{array}{c} {\dot{p}}_{6}=k_{R}U_{H}\left[p_{1}-p_{4}\right]+p_{6}\delta_{\text{IFN}}, \end{array}$$

(40) $$\begin{array}{c} {\dot{p}}_{7}=p_{2}q_{K}U_{E}+p_{3}q_{K}U_{I}+p_{7}\delta_{K}, \end{array}$$

with transversality conditions as

(41) $$\begin{array}{c} p_{i}\left(t_{f}\right)=0,\;i=1,2,3,4,5,6,7. \end{array}$$

As a result, an optimal control (*ν*) is given by

(42) $$\begin{array}{c} \nu^{*}=\max\left\{\min\left\{\frac{{U_{H}}^{*}\left[p_{1}-p_{4}\right]}{A_{3}},1\right\},0\right\}, \end{array}$$

and the optimal final time is given by

(43) $$\begin{array}{c} \frac{\partial \phi }{\partial t_{f}}\left({t_{f}}^{*}\right)=-A_{1}{U_{H}}^{*}+A_{2}{U_{R}}^{*}-\frac{A_{3}}{2}{\nu^{*}}^{2}. \end{array}$$

**Proof**

Using Pontryagin's principle, the adjoint equations and transversality conditions are obtained such that

(44) $$\begin{array}{c} {\dot{p}}_{1}=-\frac{\partial H}{\partial U_{H}}, \end{array}$$

(45) $$\begin{array}{c} {\dot{p}}_{2}=-\frac{\partial H}{\partial U_{E}}, \end{array}$$

(46) $$\begin{array}{c} {\dot{p}}_{3}=-\frac{\partial H}{\partial U_{I}}, \end{array}$$

(47) $$\begin{array}{c} {\dot{p}}_{4}=-\frac{\partial H}{\partial U_{R}}, \end{array}$$

(48) $$\begin{array}{c} {\dot{p}}_{5}=-\frac{\partial H}{\partial V}, \end{array}$$

(49) $$\begin{array}{c} {\dot{p}}_{6}=-\frac{\partial H}{\partial \left[\text{IFN}\right]}, \end{array}$$

(50) $$\begin{array}{c} {\dot{p}}_{7}=-\frac{\partial H}{\partial K}, \end{array}$$

and using the optimality conditions, the optimal control is solved as ∇_*ν*_^*H*^ = 0 in the following form:

(51) $$\begin{array}{c} A_{3}\nu +p_{1}\left(\frac{\partial {\dot{U}}_{H}}{\partial \nu }\right)+p_{2}\left(\frac{\partial {\dot{U}}_{E}}{\partial \nu }\right)+p_{3}\left(\frac{\partial {\dot{U}}_{I}}{\partial \nu }\right)+p_{4}\left(\frac{\partial {\dot{U}}_{R}}{\partial \nu }\right)+p_{5}\left(\frac{\partial \dot{V}}{\partial \nu }\right)+p_{6}\left(\frac{\partial \dot{\left[\text{IFN}\right]}}{\partial \nu }\right)+p_{7}\left(\frac{\partial \dot{K}}{\partial \nu }\right)=A_{3}\nu +p_{1}\left(-U_{H}\right)+p_{4}\left(U_{H}\right)=0. \end{array}$$

Thus, the control law is written as

(52) $$\begin{array}{c} \nu^{*}=\frac{{U_{H}}^{*}\left[p_{1}-p_{4}\right]}{A_{3}}. \end{array}$$

Using the property of the control space, the following equation is obtained:

(53) $$\begin{array}{c} \nu^{*}=\left\{\begin{array}{cc} 1 & \frac{{U_{H}}^{*}\left[p_{1}-p_{4}\right]}{A_{3}}\geq 1,\\ \frac{{U_{H}}^{*}\left[p_{1}-p_{4}\right]}{A_{3}} & 0<\frac{{U_{H}}^{*}\left[p_{1}-p_{4}\right]}{A_{3}}<1,\\ 0 & \frac{{U_{H}}^{*}\left[p_{1}-p_{4}\right]}{A_{3}}\leq 0, \end{array}\right. \end{array}$$

so, the optimal control is characterized as

(54) $$\begin{array}{c} \nu^{*}=\max\left\{\min\left\{\frac{{U_{H}}^{*}\left[p_{1}-p_{4}\right]}{A_{3}},1\right\},0\right\}. \end{array}$$

Now, according to Equation (28) and knowing *δX*_*f*_ = 0, the optimal final time (*t*_*f*_^∗^) is computed using the following equation:

(55) $$\begin{array}{c} \frac{\partial \phi }{\partial t_{f}}\left({t_{f}}^{*}\right)=-H\left({U_{H}}^{*},{U_{E}}^{*},{U_{I}}^{*},{U_{R}}^{*},V^{*},{\left[\text{IFN}\right]}^{*},K^{*},\nu^{*},{t_{f}}^{*}\right). \end{array}$$

Therefore, using the characterization of the optimal control, the following optimality system is presented to obtain the optimal control and the state. This optimal control problem consists of the state system Equations (18)–(24) with initial conditions at *t* = 0, the adjoint system Equations (34)–(40) with the final conditions Equation (41), and the characterization of the optimal control Equation (42).

(56) $$\begin{array}{c} {{\dot{U}}_{H}}^{*}=S_{H}-k_{I}{U_{H}}^{*}V^{*}-k_{R}{U_{H}}^{*}{\left[\text{IFN}\right]}^{*}-\delta_{H}{U_{H}}^{*}-\left(\max\left\{\min\left\{\frac{{U_{H}}^{*}\left[p_{1}-p_{4}\right]}{A_{3}},1\right\},0\right\}\right){U_{H}}^{*},\\ {{\dot{U}}_{E}}^{*}=k_{I}{U_{H}}^{*}V^{*}-k_{E}{U_{E}}^{*}-q_{K}{U_{E}}^{*}K^{*},\\ {{\dot{U}}_{I}}^{*}=k_{E}{U_{E}}^{*}-\delta_{I}{U_{I}}^{*}-q_{K}{U_{I}}^{*}K^{*},\\ {{\dot{U}}_{R}}^{*}=k_{R}U_{H}{\left[\text{IFN}\right]}^{*}-\delta_{R}{U_{R}}^{*}+\left(\max\left\{\min\left\{\frac{{U_{H}}^{*}\left[p_{1}-p_{4}\right]}{A_{3}},1\right\},0\right\}\right){U_{H}}^{*},\\ {\dot{V}}^{*}=\rho_{V}{U_{I}}^{*}-\delta_{V}V^{*},\\ {\dot{\left[\text{IFN}\right]}}^{*}=a_{I}{U_{I}}^{*}-\delta_{\text{IFN}}{\left[\text{IFN}\right]}^{*},\\ {\dot{K}}^{*}=S_{K}+\Phi_{K}{U_{I}}^{*}-\delta_{K}K^{*}, \end{array}$$

and the adjoint system is as follows:

(57) $$\begin{array}{c} {\dot{p}}_{1}=-A_{1}+p_{1}\delta_{H}-k_{I}V^{*}\left[p_{2}-p_{1}\right]-\left[k_{R}{\left[\text{IFN}\right]}^{*}+\max\left\{\min\left\{\frac{{U_{H}}^{*}\left[p_{1}-p_{4}\right]}{A_{3}},1\right\},0\right\}\right]\left[p_{4}-p_{1}\right],\\ {\dot{p}}_{2}=p_{2}\left[k_{E}+q_{K}K^{*}\;\right]-p_{3}k_{E},\\ {\dot{p}}_{3}=p_{3}\left[\delta_{I}+q_{K}K^{*}\;\right]-p_{5}\rho_{V}-p_{6}a_{I}-p_{7}\Phi_{K},\\ {\dot{p}}_{4}=A_{2}+p_{4}\delta_{R},\\ {\dot{p}}_{5}=k_{I}{U_{H}}^{*}\left[p_{2}+p_{1}\right]+p_{5}\rho_{V},\\ {\dot{p}}_{6}=k_{R}{U_{H}}^{*}\left[p_{1}-p_{4}\right]+p_{6}\delta_{\text{IFN}},\\ {\dot{p}}_{7}=p_{2}q_{K}{U_{E}}^{*}+p_{3}q_{K}{U_{I}}^{*}+p_{7}\delta_{K}, \end{array}$$

with *p*_1_(*t*_*f*_) = 0, *p*_2_(*t*_*f*_) = 0, *p*_3_(*t*_*f*_) = 0, *p*_4_(*t*_*f*_) = 0, *p*_5_(*t*_*f*_) = 0, *p*_6_(*t*_*f*_) = 0, *p*_7_(*t*_*f*_) = 0, *U*_*H*_(0) = *U*_*H*__0_, *U*_*E*_(0) = *U*_*E*__0_, *U*_*I*_(0) = *U*_*I*__0_, *U*_*R*_(0) = *U*_*R*__0_, *V*(0) = *V*_0_, [IFN](0) = [IFN]_0_, *K*(0) = *K*_0_, and *T*^∗^which can be rewritten as in Equation (78). So, the proof is completed.

The article "Optimal Allocation of Vaccine and Antiviral Drugs for Influenza Containment over Delayed Multiscale Epidemic Model considering Time-Dependent Transmission Rate" was published in 2021. Journal: Comput Math Methods Med.

After examining the effect of the vaccine on the person's body and the control strategy applied to the model for the best effect, it is necessary to investigate the efficiency of the optimal antiviral treatment strategy in an optimal time, which is considered in the following subsection.

### 4.2. Antiviral Treatment Strategy

This subsection is aimed at destroying the virus particles and converting healthy cells into resistant-to-infection cells simultaneously using the optimal antiviral treatment strategy. There are infected and partially infected cells within the infected individual's body. Therefore, the control input (antiviral treatment) is used to eradicate the disease by converting healthy cells to resistant-to-infection cells at the rate of *𝒯*_1_ and destroying virus particles at a rate of *𝒯*_2_.  Figure 4 shows the conceptual flow diagram of the innate immune dynamics with the proposed control action (antiviral treatment). Moreover, the dynamic of the innate immune with antiviral treatment is considered as

(58) $$\begin{array}{c} {\dot{U}}_{H}=S_{H}-k_{I}U_{H}V-k_{R}U_{H}\left[\text{IFN}\right]-\delta_{H}U_{H}-T_{1}U_{H}, \end{array}$$

(59) $$\begin{array}{c} {\dot{U}}_{E}=k_{I}U_{H}V-k_{E}U_{E}-q_{K}U_{E}K, \end{array}$$

(60) $$\begin{array}{c} {\dot{U}}_{I}=k_{E}U_{E}-\delta_{I}U_{I}-q_{K}U_{I}K, \end{array}$$

(61) $$\begin{array}{c} {\dot{U}}_{R}=k_{R}U_{H}\left[\text{IFN}\right]-\delta_{R}U_{R}+T_{1}U_{H}, \end{array}$$

(62) $$\begin{array}{c} \dot{V}=\rho_{V}U_{I}-\delta_{V}V-T_{2}V, \end{array}$$

(63) $$\begin{array}{c} \dot{\left[\text{IFN}\right]}=a_{I}U_{I}-\delta_{\text{IFN}}\left[\text{IFN}\right], \end{array}$$

(64) $$\begin{array}{c} \dot{K}=S_{K}+\Phi_{K}U_{I}-\delta_{K}K. \end{array}$$

To reach the proposed goal and minimize the cost of the optimal antiviral treatment strategy within an optimal duration, the following objective function with free terminal time has to be minimized:

(65) $$\begin{array}{c} J\left(T_{1},T_{2},t_{f}\right)=\int_{0}^{t_{f}}\left[A_{1}U_{H}-A_{2}U_{R}+A_{3}V+\frac{A_{4}}{2}{T_{1}}^{2}+\frac{A_{5}}{2}{T_{2}}^{2}\right]dt+\emptyset \left(t_{f}\right), \end{array}$$

in which *t*_*f*_ represent the duration of the antiviral treatment. ∅ is a positive increasing function such that $\underset{t⟶\infty }{\lim}\emptyset \left(t\right)=+\infty$. Also, to reach the optimal controls (*𝒯*_1_^∗^, *𝒯*_2_^∗^) and an optimal terminal time (*t*_*f*_^∗^), we considered

(66) $$\begin{array}{c} J\left({T_{1}}^{*},{T_{2}}^{*},{t_{f}}^{*}\right)=\min\left\{J\left(T_{1},T_{2},t_{f}\right)\;|\;\left(T_{1},T_{2}\right)\in U_{2},t_{f}\in {\mathbb{R}}^{+}\right\}, \end{array}$$

where *U*_2_ is the set of admissible controls defined by

(67) $$\begin{array}{c} U_{2}=\left\{\left(T_{1},T_{2}\right)\;|\;T_{1},T_{2}\right.\text{ are measurable},\;\;0\leq \left.T_{1}\leq 1,0\leq T_{2}\leq 1,t\in \left[0,t_{f}\right]\right\}. \end{array}$$

Then, the necessary conditions for optimality are written as follows:

(68) $$\begin{array}{c} \dot{p}=-\frac{\partial H}{\partial x}, \end{array}$$

(69) $$\begin{array}{c} \;{\left[\nabla_{X_{f}}^{\emptyset }-p\left(t_{f}\right)\right]}^{T}\delta X_{f}+\left[H\left(X\left(t_{f}\right),u\left(t_{f}\right),p\left(t_{f}\right),t_{f}\right)+\frac{\partial \emptyset }{\partial t_{f}}\right]{\delta t}_{f}=0, \end{array}$$

in which *t*_*f*_ is unknown while *X*(*t*_*f*_) is fixed; therefore, *δX*_*f*_ = 0. Then, the Hamiltonian for the control problem is defined as

(70) $$\begin{array}{c} H=A_{1}U_{H}-A_{2}U_{R}+A_{3}V+\frac{A_{4}}{2}{T_{1}}^{2}+\frac{A_{5}}{2}{T_{2}}^{2}+p_{1}{\dot{U}}_{H}+p_{2}{\dot{U}}_{E}+p_{3}{\dot{U}}_{I}+p_{4}{\dot{U}}_{R}+p_{5}\dot{V}+p_{6}\dot{\left[\text{IFN}\right]}+p_{7}\dot{K}, \end{array}$$

where *p*_1_, *p*_2_, *p*_3_, *p*_4_, *p*_5_, *p*_6_, and *p*_7_ are also the adjoint functions to be obtained. As discussed earlier, the following theorem is obtained to apply Pontryagin's principle to the Hamiltonian.

The article "Optimal Allocation of Vaccine and Antiviral Drugs for Influenza Containment over Delayed Multiscale Epidemic Model considering Time-Dependent Transmission Rate" was published in 2021. Journal: Comput Math Methods Med.

**Theorem 6 .**

Given optimal control pair *𝒯*_1_^∗^, *𝒯*_2_^∗^ and solutions *U*_*H*_^∗^, *U*_*E*_^∗^, *U*_*I*_^∗^, *U*_*R*_^∗^, *V*^∗^, [IFN]^∗^, and *K*^∗^ for the optimal control problem *J*(*𝒯*_1_^∗^, *𝒯*_2_^∗^, *t*_*f*_^∗^) = min{*J*(*𝒯*_1_, *𝒯*_2_, *t*_*f*_) | *𝒯*_1_, *𝒯*_2_ ∈ *U*, *t*_*f*_ ∈ ℝ^+^}, let *U*_*H*_^∗^, *U*_*E*_^∗^, *U*_*I*_^∗^, *U*_*R*_^∗^, *V*^∗^, [IFN]^∗^, and *K*^∗^ be optimal state solutions with an associated optimal control pair (*𝒯*_1_, *𝒯*_2_). There are adjoint variables that satisfy the following equations:

(71) $$\begin{array}{c} {\dot{p}}_{1}=-A_{1}+p_{1}\delta_{H}+k_{I}V\left[p_{1}-p_{2}\right]+\left[k_{R}\left[\text{IFN}\right]+\nu \right]\left[p_{1}-p_{4}\right],\\ {\dot{p}}_{2}=p_{2}\left[k_{E}+q_{K}K\;\right]-p_{3}k_{E},\\ {\dot{p}}_{3}=p_{3}\left[\delta_{I}+q_{K}K\;\right]-p_{5}\rho_{V}-p_{6}a_{I}-p_{7}\Phi_{K},\\ {\dot{p}}_{4}=A_{2}+p_{4}\delta_{R},\\ {\dot{p}}_{5}=-A_{3}+k_{I}U_{H}\left[p_{1}-p_{2}\right]+p_{4}\left[\delta_{v}+T_{2}\right],\\ {\dot{p}}_{6}=k_{R}U_{H}\left[p_{1}-p_{4}\right]+p_{6}\delta_{\text{IFN}},\\ {\dot{p}}_{7}=p_{2}q_{K}U_{E}+p_{3}q_{K}U_{I}+p_{7}\delta_{K}, \end{array}$$

with transversality conditions:

(72) $$\begin{array}{c} p_{i}\left(t_{f}\right)=0,\;\;i=1,2,3,4,5,6,7. \end{array}$$

Furthermore, the optimal controls (*𝒯*_1_, *𝒯*_2_) are given by

(73) $$\begin{array}{c} {T_{1}}^{*}=\max\left\{\min\left\{\frac{{U_{H}}^{*}\left[p_{1}-p_{4}\right]}{A_{4}},1\right\},0\right\},\\ {T_{2}}^{*}=\max\left\{\min\left\{\frac{p_{5}V^{*}}{A_{5}},1\right\},0\right\}, \end{array}$$

and the optimal final time is given by

(74) $$\begin{array}{c} \;H\left({U_{H}}^{*},{U_{E}}^{*},{U_{I}}^{*},{U_{R}}^{*},V^{*},{\left[\text{IFN}\right]}^{*},K^{*},{T_{1}}^{*},{T_{2}}^{*},{t_{f}}^{*}\right)+\frac{\partial \phi }{\partial t_{f}}\left({t_{f}}^{*}\right)=0. \end{array}$$

**Proof**

The adjoint equation and transversality conditions can be obtained using Pontryagin's principle as similar to Equations (44)–(50). Then, by using the optimality conditions, the optimal controls are obtained using ∇_*𝒯*_1__^*H*^ = 0 and ∇_*𝒯*_2__^*H*^ = 0. As a result, the control inputs are computed as

(75) $$\begin{array}{c} {T_{1}}^{*}=\frac{{U_{H}}^{*}\left[p_{1}-p_{4}\right]}{A_{3}},\\ {T_{2}}^{*}=\frac{p_{5}V^{*}}{A_{5}}. \end{array}$$

Using the property of the control space, we obtain

(76) $$\begin{array}{c} {T_{1}}^{*}=\left\{\begin{array}{cc} 1 & \frac{{U_{H}}^{*}\left[p_{1}-p_{4}\right]}{A_{4}}\geq 1,\\ \frac{{U_{H}}^{*}\left[p_{1}-p_{4}\right]}{A_{3}} & 0<\frac{{U_{H}}^{*}\left[p_{1}-p_{4}\right]}{A_{4}}<1,\\ 0 & \frac{{U_{H}}^{*}\left[p_{1}-p_{4}\right]}{A_{4}}\leq 0, \end{array}\right.\\ {T_{2}}^{*}=\left\{\begin{array}{cc} 1 & \frac{p_{5}V^{*}}{A_{5}}\geq 1,\\ \frac{p_{5}V^{*}}{A_{5}} & 0<\frac{p_{5}V^{*}}{A_{5}}<1,\\ 0 & \frac{p_{5}V^{*}}{A_{5}}\leq 0. \end{array}\right. \end{array}$$

So, the optimal control is characterized as

(77) $$\begin{array}{c} {T_{1}}^{*}=\max\left\{\min\left\{\frac{{U_{H}}^{*}\left[p_{1}-p_{4}\right]}{A_{4}},1\right\},0\right\},\\ {T_{2}}^{*}=\max\left\{\min\left\{\frac{p_{5}V^{*}}{A_{5}},1\right\},0\right\}, \end{array}$$

and according to Equation (74) and knowing that *δX*_*f*_ = 0, the optimal final time (*t*_*f*_^∗^) is computed using the following equation:

(78) $$\begin{array}{c} \;\frac{\partial \phi }{\partial t_{f}}\left({t_{f}}^{*}\right)=-A_{1}{U_{H}}^{*}-A_{2}{U_{R}}^{*}+A_{3}V^{*}+\frac{A_{4}}{2}{{T_{1}}^{*}}^{2}+\frac{A_{5}}{2}{{T_{2}}^{*}}^{2}. \end{array}$$

Therefore, using the characterization of the optimal control, we have the following optimality system to obtain the optimal states:

(79) $$\begin{array}{c} {{\dot{U}}_{H}}^{*}=S_{H}-k_{I}{U_{H}}^{*}V^{*}-k_{R}{U_{H}}^{*}{\left[\text{IFN}\right]}^{*}-\delta_{H}{U_{H}}^{*}-\left(\max\left\{\min\left\{\frac{{U_{H}}^{*}\left[p_{1}-p_{4}\right]}{A_{4}},1\right\},0\right\}\right){U_{H}}^{*},\\ {{\dot{U}}_{E}}^{*}=k_{I}{U_{H}}^{*}V^{*}-k_{E}{U_{E}}^{*}-q_{K}{U_{E}}^{*}K^{*},\\ {{\dot{U}}_{I}}^{*}=k_{E}{U_{E}}^{*}-\delta_{I}{U_{I}}^{*}-q_{K}{U_{I}}^{*}K^{*},\\ {{\dot{U}}_{R}}^{*}=k_{R}U_{H}{\left[\text{IFN}\right]}^{*}-\delta_{R}{U_{R}}^{*}+\left(\max\left\{\min\left\{\frac{{U_{H}}^{*}\left[p_{1}-p_{4}\right]}{A_{4}},1\right\},0\right\}\right){U_{H}}^{*},\\ {\dot{V}}^{*}=\rho_{V}{U_{I}}^{*}-\delta_{V}V^{*}-\max\left\{\min\left\{\frac{p_{5}V^{*}}{A_{5}},1\right\},0\right\}V^{*},\\ {\dot{\left[\text{IFN}\right]}}^{*}=a_{I}{U_{I}}^{*}-\delta_{\text{IFN}}{\left[\text{IFN}\right]}^{*},\\ {\dot{K}}^{*}=S_{K}+\Phi_{K}{U_{I}}^{*}-\delta_{K}K^{*}, \end{array}$$

and the adjoint equations are as follows:

(80) $$\begin{array}{c} {\dot{p}}_{1}=-A_{1}+p_{1}\delta_{H}-k_{I}V^{*}\left[p_{2}-p_{1}\right]-\left[k_{R}{\left[\text{IFN}\right]}^{*}+\max\left\{\min\left\{\frac{{U_{H}}^{*}\left[p_{1}-p_{4}\right]}{A_{4}},1\right\},0\right\}\right]\left[p_{4}-p_{1}\right],\\ {\dot{p}}_{2}=p_{2}\left[k_{E}+q_{K}K^{*}\;\right]-p_{3}k_{E},\\ {\dot{p}}_{3}=p_{3}\left[\delta_{I}+q_{K}K^{*}\;\right]-p_{5}\rho_{V}-p_{6}a_{I}-p_{7}\Phi_{K},\\ {\dot{p}}_{4}=A_{2}+p_{4}\delta_{R},\\ {\dot{p}}_{5}=-A_{3}+k_{I}{U_{H}}^{*}\left[p_{1}-p_{2}\right]+p_{4}\left[\delta_{v}+\max\left\{\min\left\{\frac{p_{5}V^{*}}{A_{5}},1\right\},0\right\}\right],\\ {\dot{p}}_{6}=k_{R}{U_{H}}^{*}\left[p_{1}-p_{4}\right]+p_{6}\delta_{\text{IFN}},\\ {\dot{p}}_{7}=p_{2}q_{K}{U_{E}}^{*}+p_{3}q_{K}{U_{I}}^{*}+p_{7}\delta_{K}, \end{array}$$

where *p*_1_(*t*_*f*_) = 0, *p*_2_(*t*_*f*_) = 0, *p*_3_(*t*_*f*_) = 0, *p*_4_(*t*_*f*_) = 0, *p*_5_(*t*_*f*_) = 0, *p*_6_(*t*_*f*_) = 0, *p*_7_(*t*_*f*_) = 0, *U*_*H*_(0) = *U*_*H*__0_, *U*_*E*_(0) = *U*_*E*__0_, *U*_*I*_(0) = *U*_*I*__0_, *U*_*R*_(0) = *U*_*R*__0_, *V*(0) = *V*_0_, [IFN](0) = [IFN]_0_, and *K*(0) = *K*_0_. Then, the proof is completed.

The article "Optimal Allocation of Vaccine and Antiviral Drugs for Influenza Containment over Delayed Multiscale Epidemic Model considering Time-Dependent Transmission Rate" was published in 2021. Journal: Comput Math Methods Med.

**Remark 1 .**

In the vaccination strategy, the healthy cells convert to resistant-to-infection cells using the proposed controller and their number converges to zero when *t*⟶∞(*U*_*H*_⟶0) and the rest remain at their initial zero value, while in the antiviral treatment strategy, in addition to converting healthy cells to resistant-to-infection cells, the virus particles decrease and converge to zero using the proposed controller. Meanwhile, the number of natural killers converges to the initial constant value. Then, after a while, Equation (59) becomes ${\dot{U}}_{E}=-\left(k_{E}+q_{K}K\right)U_{E}$ in which (*k*_*E*_ + *q*_*K*_*K*) is constant and is considered as first-order linear differential equation that yields *U*_*E*_ = *U*_*E*__0_*e*^−(*k*_*E*_ + *q*_*K*_*K*)*t*^. As a result, *U*_*E*_ converges exponentially to zero.

In this section, the effect of the optimal control on the within-host model is examined. At the same time, it is necessary to explore the controller's influence on the between-hosts model (SEIR epidemic model). Thus, the impact of the delay computed in this section is discussed in the following section in detail.

## 5. SEIR Dynamic Model

In this section, a SEIR epidemic model is introduced with two additional properties. First is two time-delay that aroused from this fact that vaccination and antiviral treatment take time to impact a person's body. Second is a nonlinear contact rate (transmission rate) function that is followed by this fact that the contact rate is varying throughout day and night. In this regard, the susceptible and infected individuals move to the recovered people group with time delays *t*_1_ and *t*_2_ (optimal times of vaccination and antiviral treatment within the body, which is computed in the previous section), respectively. The proposed SEIR epidemic model is presented as

(81) $$\begin{array}{c} \dot{S}\left(t\right)=-\beta \left(t\right)S\left(t\right)I\left(t\right)+\mu_{d}\left(3\left(1-\rho I\left(t\right)\right)-S\left(t\right)\right),\\ \dot{E}\left(t\right)=\beta \left(t\right)S\left(t\right)I\left(t\right)-\left(\mu_{d}+\kappa \right)E\left(t\right),\\ \dot{I}\left(t\right)=\kappa E\left(t\right)-\alpha I\left(t\right),\\ \dot{R}\left(t\right)=gI\left(t\right)-\mu_{d}R\left(t\right), \end{array}$$

where *α* = (*g* − 3*μ*_*d*_*ρ* + *μ*_*d*_). As shown in Figure 5, *S*(*t*) represents the number of susceptible individuals who are vulnerable and not infected, *E*(*t*) or exposed individual denotes the number of people that are infected but not infectious yet, *I*(*t*) signifies the population of infectious people with symptoms that can transmit the disease to others, and *R*(*t*) is the number of completely recovered (immune) people. *N* is the total population size (*S*(*t*) + *E*(*t*) + *I*(*t*) + *R*(*t*) = *N*). *μ*_*d*_ is the rate of deaths from causes unrelated to the infection, and *μ*_*b*_ is the birth rate in each group, which is triple the mortality rate (*μ*_*b*_ = 3*μ*_*d*_). *t*_1_ is the vaccination time of susceptible people, and *t*_2_ is the recovery time of infected people. In the case of births, in the susceptible, exposed, and recovered groups, newborns are susceptible to the disease and add to the susceptible group at the rate of *μ*_*b*_. Fraction *ρ* of the infected individuals' infants goes to the infected compartment, and the others (fraction (1 − *ρ*) of infected individuals' infants) move to the susceptible group. The exposed people get infected at a rate of *κ*, and infected people leave their compartment at the rate of *α*.

The article "Optimal Allocation of Vaccine and Antiviral Drugs for Influenza Containment over Delayed Multiscale Epidemic Model considering Time-Dependent Transmission Rate" was published in 2021. Journal: Comput Math Methods Med.

The contact rate is *β*(*t*) that is purposefully variable throughout day and night. It is also obvious that this rate at night is higher than during the day, which makes it closer to the real world and is more effective in practice [40]. According to the basic definition of *β*(*t*) that is defined as “the average number of contacts between individuals in the population per unit time” [40], the contact rate must be more than one during the day due to the more relations between people in the community. Moreover, late at night and early in the morning, the transmission rate is less than one. Therefore, with trial and error and taking into account the assumptions below, the contact rate is obtained as *β*(*t*) = 0.5(3 − sin(2*πt*)^2^ − sin(2*πt*) − cos(2*πt*)).

- 00:00 midnight: *β*(00 : 00) = 1
- 06:00 morning: *β*(06 : 00) = 0.5
- 12:00 midday: *β*(12 : 00) = 2
- 18:00 evening: *β*(18 : 00) = 1.5

Thus, the contact rate is less than one late at night and at daybreak and is greater than one in the middle of the day because there are more social gatherings and offices and schools are also open.

In the next section, an optimal control is applied to the proposed model to overcome the disease outbreak.

## 6. Optimal Control of the Between-Hosts Epidemic Model

The aim of this section is twofold: first, minimizing the number of susceptible individuals and moving them to the recovered group by vaccination at a rate of *u*_*v*_(0 ≤ *u*_*v*_ ≤ 1) in 25 days and second, moving the infected people to the recovered group at a rate of *u*_*τ*_(0 ≤ *u*_*τ*_ ≤ 1) by antiviral treatment in 25 days, as shown in Figure 5. The SEIR dynamic model in the presence of the controller is presented as

(82) $$\begin{array}{c} \dot{S}\left(t\right)=-\beta \left(t\right)S\left(t\right)I\left(t\right)+\mu_{d}\left(3\left(1-\rho I\left(t\right)\right)-S\left(t\right)\right)-u_{v}\left(t-t_{1}\right)S\left(t\right), \end{array}$$

(83) $$\begin{array}{c} \dot{E}\left(t\right)=\beta \left(t\right)S\left(t\right)I\left(t\right)-\left(\mu_{d}+\kappa \right)E\left(t\right), \end{array}$$

(84) $$\begin{array}{c} \dot{I}\left(t\right)=\kappa E\left(t\right)-\alpha I\left(t\right)-u_{\tau }\left(t-t_{2}\right)I\left(t\right), \end{array}$$

(85) $$\begin{array}{c} \dot{R}\left(t\right)=gI\left(t\right)-\mu_{d}R\left(t\right)+u_{v}\left(t-t_{1}\right)S\left(t\right)+u_{\tau }\left(t-t_{2}\right)I\left(t\right), \end{array}$$

where *u*_*v*_(*t*) = 0 for *t* ∈ [−*t*_1_, 0] and *u*_*τ*_(*t*) = 0 for *t* ∈ [−*t*_2_, 0].

The article "Optimal Allocation of Vaccine and Antiviral Drugs for Influenza Containment over Delayed Multiscale Epidemic Model considering Time-Dependent Transmission Rate" was published in 2021. Journal: Comput Math Methods Med.

To this end, the optimal control strategy is used to achieve these goals. The objective function is considered as

(86) $$\begin{array}{c} J\left(u_{v}\left(t\right),u_{\tau }\left(t\right),t_{f}\right)=\int_{0}^{t_{f}}\left[B_{1}I\left(t\right)+B_{2}S\left(t\right)-B_{3}R\left(t\right)+\frac{B_{4}}{2}u_{v}{\left(t\right)}^{2}+\frac{B_{5}}{2}u_{\tau }{\left(t\right)}^{2}\right]dt, \end{array}$$

where *B*_1_, *B*_2_, and *B*_3_ are gains of the infected, susceptible, and recovered individuals. Also, *B*_4_ and *B*_5_ are the gains of control inputs *u*_*v*_, and *u*_*τ*_, respectively. Moreover, *t*_*f*_ and *X*(*t*_*f*_) are fixed. Tacking the Hamiltonian yields

(87) $$\begin{array}{c} H=B_{1}I\left(t\right)+B_{2}S\left(t\right)-B_{3}R\left(t\right)+\frac{B_{4}}{2}u_{v}{\left(t\right)}^{2}+\frac{B_{5}}{2}u_{\tau }{\left(t\right)}^{2}+p_{1}\dot{S}\left(t\right)+p_{2}\dot{E}\left(t\right)+p_{3}\dot{I}\left(t\right)+p_{4}\dot{R}\left(t\right), \end{array}$$

where *p*_1_.*p*_2_, *p*_3_, and *p*_4_ are adjoint functions that satisfy the adjoint equations. Pontryagin's maximum principle is applied to the Hamiltonian *H* to derive the necessary conditions for the optimal control. The adjoint equation and transversality conditions are obtained by using Pontryagin's maximum principle such that

(88) $$\begin{array}{c} {\dot{p}}_{1}=-\frac{\partial H}{\partial S\left(t\right)}=-B_{2}+\beta \left(t\right)I\left(t\right)\left[p_{1}-p_{2}\right]+u_{v}\left(t-t_{1}\right)\left[p_{1}-p_{4}\right]+p_{1}\mu_{d},p_{1}\left(t_{f}\right)=0,\\ {\dot{p}}_{2}=-\frac{\partial H}{\partial E\left(t\right)}=\kappa \;\left(p_{2}-p_{3}\right)+p_{2}\mu_{d},p_{2}\left(t_{f}\right)=0,\\ {\dot{p}}_{3}=-\frac{\partial H}{\partial I\left(t\right)}=-B_{1}+\beta \left(t\right)S\left(t\right)\left[p_{1}-p_{2}\right]+u_{\tau }\left(t-t_{2}\right)\left[p_{3}-p_{4}\right]+p_{3}\alpha -p_{4}g,p_{3}\left(t_{f}\right)=0,\\ {\dot{p}}_{4}=-\frac{\partial H}{\partial R\left(t\right)}=B_{3}+p_{4}\mu_{d},p_{4}\left(t_{f}\right)=0. \end{array}$$

Notice that the control *u*_*v*_(*t* − *t*_1_) can only influence the state variable on the time interval [*t*_*f*_ − *t*_1_, *t*_*f*_]. Thus, it suffices to compute the optimal control on the interval [0, *t*_*f*_ − *t*_1_]. Therefore, we have

(89) $$\begin{array}{c} \frac{\partial H}{\partial u_{v}\left(t\right)}+{\left.\frac{\partial H}{\partial u_{v}\left(t-t_{1}\right)}\right|}_{t+t_{1}}=0, \end{array}$$

which yields

(90) $$\begin{array}{c} \left\{\begin{array}{cc} {u_{v}}^{*}\left(t\right)=\frac{S^{*}\left(t+t_{1}\right)\left[p_{1}\left(t+t_{1}\right)-p_{4}\left(t+t_{1}\right)\right]}{B_{4}}, & t\in \left[0,t_{f}-t_{1}\right],\\ {u_{v}}^{*}\left(t\right)=0, & t\in \left[t_{f}-t_{1},t_{f}\right]. \end{array}\right. \end{array}$$

Similarly,

(91) $$\begin{array}{c} \frac{\partial H}{\partial u_{\tau }\left(t\right)}+{\left.\frac{\partial H}{\partial u_{\tau }\left(t-t_{2}\right)}\right|}_{t+t_{2}}=0 \end{array}$$

that can be written as

(92) $$\begin{array}{c} \left\{\begin{array}{cc} {u_{\tau }}^{*}\left(t\right)=\frac{I^{*}\left(t+t_{2}\right)\left[p_{3}\left(t+t_{2}\right)-p_{4}\left(t+t_{2}\right)\right]}{B_{5}}, & t\in \left[0,t_{f}-t_{2}\right],\\ {u_{\tau }}^{*}\left(t\right)=0, & t\in \left[t_{f}-t_{2},t_{f}\right], \end{array}\right. \end{array}$$

which yields

(93) $$\begin{array}{c} {u_{v}}^{*}\left(t\right)=\left\{\begin{array}{cc} 1 & \frac{S^{*}\left(t+t_{1}\right)\left[p_{1}\left(t+t_{1}\right)-p_{4}\left(t+t_{1}\right)\right]}{B_{4}}\geq 1,\\ \frac{S^{*}\left(t+t_{1}\right)\left[p_{1}\left(t+t_{1}\right)-p_{4}\left(t+t_{1}\right)\right]}{B_{4}} & 0<\frac{S^{*}\left(t+t_{1}\right)\left[p_{1}\left(t+t_{1}\right)-p_{4}\left(t+t_{1}\right)\right]}{B_{4}}<1,\\ 0 & \frac{S^{*}\left(t+t_{1}\right)\left[p_{1}\left(t+t_{1}\right)-p_{4}\left(t+t_{1}\right)\right]}{B_{4}}\leq 0, \end{array}\right.\\ {u_{\tau }}^{*}\left(t\right)=\left\{\begin{array}{cc} 1 & \frac{I^{*}\left(t+t_{2}\right)\left[p_{3}\left(t+t_{2}\right)-p_{4}\left(t+t_{2}\right)\right]}{B_{5}}\geq 1,\\ \frac{I^{*}\left(t+t_{2}\right)\left[p_{3}\left(t+t_{2}\right)-p_{4}\left(t+t_{2}\right)\right]}{B_{5}} & 0<\frac{I^{*}\left(t+t_{2}\right)\left[p_{3}\left(t+t_{2}\right)-p_{4}\left(t+t_{2}\right)\right]}{B_{5}}<1,\\ 0 & \frac{I^{*}\left(t+t_{2}\right)\left[p_{3}\left(t+t_{2}\right)-p_{4}\left(t+t_{2}\right)\right]}{B_{5}}\leq 0. \end{array}\right. \end{array}$$

So, the optimal controls are given as

(94) $$\begin{array}{c} {u_{v}}^{*}\left(t\right)=\max\left\{\min\left\{\frac{S^{*}\left(t+t_{1}\right)\left[p_{1}\left(t+t_{1}\right)-p_{4}\left(t+t_{1}\right)\right]}{B_{4}},1\right\},0\right\},\;t\in \left[0,t_{f}-t_{1}\right],\\ {u_{\tau }}^{*}\left(t\right)=\max\left\{\min\left\{\frac{I^{*}\left(t+t_{2}\right)\left[p_{3}\left(t+t_{2}\right)-p_{4}\left(t+t_{2}\right)\right]}{B_{5}},1\right\},0\right\},\;t\in \left[0,t_{f}-t_{2}\right]. \end{array}$$

Therefore, using the characterization of the optimal control and considering Equations (90) and (92), the following optimality system is obtained as

(95) $$\begin{array}{c} {\dot{S}}^{*}\left(t\right)=-\beta \left(t\right)S^{*}\left(t\right)I^{*}\left(t\right)+\mu_{d}\left(3\left(1-\rho I^{*}\left(t\right)\right)-S^{*}\left(t\right)\right)-{u_{v}}^{*}\left(t\right)S^{*}\left(t\right),\\ {\dot{E}}^{*}\left(t\right)=\beta \left(t\right)S^{*}\left(t\right)I^{*}\left(t\right)-\left(\mu_{d}+\kappa \right)E^{*}\left(t\right),\\ {\dot{I}}^{*}\left(t\right)=\kappa E^{*}\left(t\right)-gI^{*}\left(t\right)-{u_{\tau }}^{*}\left(t\right)I^{*}\left(t\right),\\ {\dot{R}}^{*}\left(t\right)=gI^{*}\left(t\right)-\mu_{d}R^{*}\left(t\right)+{u_{v}}^{*}\left(t\right)S^{*}\left(t\right)+{u_{\tau }}^{*}\left(t\right)I^{*}\left(t\right). \end{array}$$

The adjoint equations are also obtained as

(96) $$\begin{array}{c} {\dot{p}}_{1}=-B_{2}+\beta \left(t\right)I^{*}\left(t\right)\left[p_{1}-p_{2}\right]+u_{v}^{*}\left(t-t_{1}\right)\left[p_{1}-p_{4}\right]+p_{1}\mu_{d},\\ {\dot{p}}_{2}=\kappa \;\left(p_{2}-p_{3}\right)+p_{2}\mu_{d},\\ {\dot{p}}_{3}=-B_{1}+\beta \left(t\right)S^{*}\left(t\right)\left[p_{1}-p_{2}\right]+u_{\tau }^{*}\left(t-t_{2}\right)\left[p_{3}-p_{4}\right]+p_{3}\alpha -p_{4}g,\\ {\dot{p}}_{4}=B_{3}+p_{4}\mu_{d}, \end{array}$$

where *p*_1_(*t*_*f*_) = 0, *p*_2_(*t*_*f*_) = 0, *p*_3_(*t*_*f*_) = 0, *p*_4_(*t*_*f*_) = 0, *p*_5_(*t*_*f*_) = 0, *p*_6_(*t*_*f*_) = 0, *p*_7_(*t*_*f*_) = 0, *S*(0) = *S*_0_, *E*(0) = *E*_0_, *I*(0) = *I*_0_, and *R*(0) = *R*_0_.

The article "Optimal Allocation of Vaccine and Antiviral Drugs for Influenza Containment over Delayed Multiscale Epidemic Model considering Time-Dependent Transmission Rate" was published in 2021. Journal: Comput Math Methods Med.

**Remark 2 .**

According to the proposed controller, susceptible and infected persons converge to zero as ⟶∞(*S*(*t*), *I*(*t*)⟶0); then, Equation (83) becomes a first-order linear differential equation as $\dot{E}\left(t\right)=-\left(\mu_{d}+\kappa \right)E\left(t\right)$ in which (*μ*_*d*_ + *κ*) is a positive constant and yields *E*(*t*) = *E*_0_*e*^−(*μ*_*d*_ + *κ*)*t*^. Thereupon, *E*(*t*) converges exponentially to zero indirectly and as a result of zeroing infected and susceptible people.

After investigating the effect of the proposed controller on both models, the results of the controller actions should be illustrated. Therefore, the simulation results of the proposed work are outlined in the next section.

## 7. Simulation Results

In this section, a numerical simulation is given to prove the accuracy of the results obtained in the previous sections. First, the effect of the optimal controllers on the innate immune response and then on the SEIR epidemic model is assessed. The value of innate immune response parameters (*k*_*I*_, *k*_*R*_, *k*_*E*_, *q*_*K*_, *Φ*_*K*_, *a*_*I*_, *ρ*_*V*_, *δ*_*H*_, *δ*_*I*_, *δ*_*R*_, *δ*_IFN_, *δ*_*K*_, *δ*_*V*_, *S*_*H*_, *S*_*K*_) is based on experimental data from Hernandez-Vargas and Meyer-Hermann [7], and the parameter values of the SEIR epidemic model are *κ* = *g* = *ρ* = 0.3 and *μ*_*d*_ = 0.02. The initial values of the SEIR epidemic model states and innate immune response model are shown in Tables 2 and 3, respectively.

This section is categorized as follows:

(a) The influence of model parameters
(b) The effect of the optimal controller on the within-host model. This section is divided into the following two subsections:
  - Within-host vaccination
  - Within-host therapy
(c) The effect of the optimal controller on the between-hosts model. This section is divided into the following two subsections:
  - Between-hosts vaccination
  - Between-hosts therapy

### 7.1. Influence of Model Parameters

This section is aimed at conducting the sensitivity analysis to identify the factors that noticeably affect the number of people engaged in influenza. Therefore, the changes in the value of parameters *β*(*t*), *g*, and *k* are investigated, respectively. The tremendous influence of contact rate cannot be neglected. The susceptible people get infected if they have more contact with infected people; as a result, the epidemic widely spreads. Thus, the contact rate has to be considered as a critical parameter in the epidemic containment process. To this end, the value of the contact rate is changed from 0.6 *β*(*t*) to 1.4 *β*(*t*) to observe its impact on the population size in each engaged group. As shown in Figures 6(a)–6(d), by increasing in the value of contact rate to 1.4 *β*(*t*), as a result, the more contact between people, the number of susceptible people reduces regarding increment in the number of infected people, while the number of susceptible people does not decrease more because of the less contact between infected individuals (0.6 *β*(*t*)). Obviously, the number of exposed and infected people decreases followed by nearly half decrement in the contact rate with susceptible people. Thus, few people get infected; as a result, few people have recovered.

The article "Optimal Allocation of Vaccine and Antiviral Drugs for Influenza Containment over Delayed Multiscale Epidemic Model considering Time-Dependent Transmission Rate" was published in 2021. Journal: Comput Math Methods Med.

In Figure 7, the impact of changes in the value of *g*, which is the recovery rate of infected people, is presented. As shown in Figure 7(a), when the rate of *g* is doubled, a greater number of susceptible people have recovered; as a result, fewer people get infected and the number of susceptible people is increased. Moreover, the number of infected people increases when the recovery rate decreases and decreases with increment in the value of recovery rate because more infected people are recovered. As a result, it is obvious that the number of recovered people is grown up followed by the rise in the recovery rate.

According to Figure 8, the exposed people are infected at a rate of *κ*; therefore, increment in this rate leads to growth in the infected people number; as a result, there is growth in the number of recovered people. It is obvious that the number of susceptible people is decreased when *κ* increases.

As observed, for different values of *β*(*t*), *g*, and *k*, the disease does not disappear in about 25 days; therefore, it is necessary to use vaccination and antiviral treatment strategies to overcome the epidemic. Thus, in the next sections, the model in the presence of vaccination and antiviral treatment is simulated compared to the model without the controller.

### 7.2. Optimal Control Results in the Within-Host Model

In the real world, susceptible people will not immediately become immune to the infection following vaccination because it takes time for all healthy cells (within the susceptible individual's body) to become resistant-to-infection cells. Moreover, the destruction of the virus (and at the same time the transformation of healthy cells into resistant-to-infection cells) within the infected person's body is not immediate with antiviral therapy; therefore, the infected person is treated after a while. To this end, two-time delay (the length of vaccination and antiviral treatment) is considered in the SEIR model.

#### 7.2.1. Within-Host Vaccination

Vaccine injection into the susceptible individual's body makes the healthy cells resistant-to-infection. Consequently, the susceptible individual, which includes healthy cells, will be recovered against the infection. Converting the healthy cells into the resistant-to-infection cells takes time, which is considered as delay in recovering process of susceptible individuals in the SEIR model. In Section 4, initially, the optimal time of healthy cells converting into resistant-to-infection cells in the susceptible individual's body has been obtained. Numerical simulations suggest eight days as the optimal time to convert the healthy cells into the resistant ones in a susceptible person's body (see Figure 9). The proposed optimal time will be considered as a delay of moving susceptible people to the recovered people group in the SEIR model in the next section.

The article "Optimal Allocation of Vaccine and Antiviral Drugs for Influenza Containment over Delayed Multiscale Epidemic Model considering Time-Dependent Transmission Rate" was published in 2021. Journal: Comput Math Methods Med.

Figures 10(a) and 10(b) show the effect of control input (vaccination) on the number of healthy and resistant-to-infection cells. There is a surge in the number of resistant-to-infection cells during vaccination in eight days. After vaccination, it can be deduced that rising in the resistant-to-infection cell numbers is associated with the reduction in the healthy cell numbers, indicating the controller efficacy. As mentioned, as the number of resistant-to-infection cells increases moment by moment, the susceptible person eventually becomes immune to the disease after eight days because the healthy cells in his/her body have all become resistant.

#### 7.2.2. Within-Host Therapy

There are virus particles (as a result, infected and partially infected cells) in the infected person's body. Therefore, the infected person needs to be treated with antiviral treatment. Thus, over the treatment process, the infected and partially infected cells and virus particles are killed, and the healthy cells become resistant-to-infection simultaneously, which also takes time.

In Figure 11, the final optimal time to eradicate disease computed in Section 4 is shown. As shown in Figures 12(a) and 12(b), using antiviral drugs, healthy cells become resistant-to-infection cells. The drug's effect on infected and partially infected cells and viruses can also be seen in Figures 13 and 14, respectively. It is clear that the infected and partially infected cells are destroyed within six days, and the number of virus particles is also converged to zero, which indicates that the infected person is cured. Moreover, the evolution of IFN-I molecules and natural killer cells with and without the controller is shown in Figures 15(a) and 15(b).

### 7.3. Optimal Control Results between Hosts

In this section, we examine the effect of the optimal controller on the SEIR epidemic model, which was discussed in Section 7, in detail. First, the changes in the number of susceptible, exposed, infected, and recovered individuals in the absence of appropriate control are investigated. Then, the effect of the vaccination strategy and antiviral treatment on individuals in a community is examined. For the numerical simulations, the delay differential equation solver (dde23) is used. This solver does not solve the advance equations (*t* + *t*_*i*_) directly; therefore, it is necessary to convert the advance equations into delay differential equations. To this end, a new reversed-time variable *ς* = *t*_*f*_ − *t* is defined and new adjoint variables *λ*_*i*_(*ς*) = *p*_*i*_(*t*_*f*_ − *ς*) are introduced. Thus, this new system is solved numerically using dde23.

The article "Optimal Allocation of Vaccine and Antiviral Drugs for Influenza Containment over Delayed Multiscale Epidemic Model considering Time-Dependent Transmission Rate" was published in 2021. Journal: Comput Math Methods Med.

#### 7.3.1. Between-Hosts Vaccination

As shown in Figures 16(a) and 16(b), the number of susceptible individuals in the absence of a controller (vaccination has not been applied) descends and converts to infected people. Eventually, it remains stationary at a constant value (less than 2,000 people). Besides, the number of recovered people without any controller is greater than their number in the control-based strategy. The number of recovered people has reached more than 10,000 because in the absence of effective treatment, more people become infected, and as a result, more people will be recovered. By injecting the vaccine into the susceptible person's body, during the conversion of healthy cells to resistant cells, the susceptible person also vaccinates (direct transfer of individuals from the susceptible group to the recovered group). As a result, the number of susceptible individuals decreases and moves to the recovered individual group at the same time. This means the susceptible people vaccinate against the disease in almost 25 days (*t*_3_) (the healthy cells of the susceptible individual convert to resistant-to-infection cells in eight days as the delay time with vaccination), while in [13], the final time of the vaccination campaign of nearly 40 days is suggested without considering the delay in the vaccination of susceptible people.

#### 7.3.2. Between-Hosts Therapy

When the infection spreads in the community without control over its prevalence, the number of infected people is increasing every day, as shown in Figure 17(a). It rose by over 3,000 people. Finally, their number decreases until the 25^th^ day and reaches a little under 2,000 and remains unchanged, indicating the community's disease persistence. Also, the exposed people number reaches a high number of 4,000 in only twelve days and ultimately converges to a stable population and remains at almost 1,500 (see Figure 17(b)).

In contrast, the number of infected people exceeds almost 500 with antiviral therapy, which is used to treat infected people (transfer them to a recovered group). During the computed optimal time (the same delay as six days), the healthy cells convert to resistant-to-infection cells; at the same time, virus particles are eradicated by antiviral treatment in the infected person's body. Therefore, the infected people move to the recovered people group in almost 25 days. According to Remark 8, the number of exposed people also converges to zero as a result of decrement of infected people in 25 days.

The article "Optimal Allocation of Vaccine and Antiviral Drugs for Influenza Containment over Delayed Multiscale Epidemic Model considering Time-Dependent Transmission Rate" was published in 2021. Journal: Comput Math Methods Med.

## 8. Conclusion

In this paper, the optimal control theory was applied to two types of dynamic epidemic models: the innate immune response dynamic and the SEIR epidemic model. A nonlinear transmission rate and time delay were considered in the SEIR epidemic model. The aim of this paper was twofold: firstly, preventing the virus from spreading within the body of a host and secondly, curb the epidemic in the society and between hosts. To this end, two control strategies were introduced to satisfy the first goal in the susceptible and infected person's bodies. In this regard, vaccination was used to convert healthy cells to resistant-to-infection cells inside the susceptible individual's body that recovered them against the disease in society. In the following, antiviral treatment was used to reduce the concentration of viruses and convert healthy cells to resistant-to-infection cells at the same time inside the infected individual's body to recover them. Moreover, to control the epidemic in society, the optimal control was used to increase the number of recovered people by reducing the number of susceptible and infected people in the fixed 25 days. Transferring occurred with a delay computed as the optimal time of disease eradication inside the infected individual's body and the recovery of the susceptible individual's body. Finally, numerical simulation was used to illustrate the usefulness of the obtained results.

## Figures and Tables

**Figure 1:** Block diagram of the relationship between innate immune response and SEIR model.

**Figure 2:** The disease modeling with two scales: within a host and between hosts.

**Figure 3:** Conceptual flow diagram of innate immune dynamics with vaccination.

**Figure 4:** The diagram of the innate immune dynamics with the proposed control action (antiviral treatment).

**Figure 5:** Conceptual flow diagram of the influenza SEIAR dynamics with the proposed controllers.

**Figure 6:** The impact of the contact rate changes on the (a) susceptible, (b) exposed, (c) infected, and (d) recovered people.

**Figure 7:** The impact of the recovery rate changes on the (a) susceptible, (b) exposed, (c) infected, and (d) recovered people.

**Figure 8:** The impact of the *κ* rate changes on the (a) susceptible, (b) exposed, (c) infected, and (d) recovered people.

**Figure 9:** The optimal final time.

**Figure 10:** Evolution of healthy cells and resistant-to-infection cells with and without the controller.

The article "Optimal Allocation of Vaccine and Antiviral Drugs for Influenza Containment over Delayed Multiscale Epidemic Model considering Time-Dependent Transmission Rate" was published in 2021. Journal: Comput Math Methods Med.

**Figure 11:** The optimal final time.

**Figure 12:** Evolution of healthy cells and resistant-to-infection cells with and without the controller.

**Figure 13:** Evolution of partially infected cells and infected cells with and without the controller.

**Figure 14:** Evolution of virus particle with and without the controller.

**Figure 15:** Evolution of IFN-I molecules and natural killer cells with and without the controller.

**Figure 16:** The population of susceptible and recovered individuals with and without the controller.

**Figure 17:** The population of infected and exposed individuals with and without the controller.

**Algorithm 1:** General strategy algorithm.

**Table 1:** Equilibrium values of the model.

State variable	DFE	EE
${\bar{U}}_{H}$	$\frac{S_{H}}{\delta_{H}}$	2.44 × 10^6^
${\bar{U}}_{E}$	0	8.94 × 10^5^
${\bar{U}}_{I}$	0	1.84 × 10^5^
${\bar{U}}_{R}$	0	2.37 × 10^8^
$\bar{V}$	0	354.65
$\left[\bar{IFN}\right]$	0	0.138
$\bar{K}$	$\frac{S_{K}}{\delta_{K}}$	804.610 × 10^3^

**Table 2:** Initial values of the SEIR epidemic model.

State variable	Initial value
**S**_0_	9375
**E**_0_	125
**I**_0_	313
**R**_0_	0
**N**_0_	10,000

**Table 3:** Initial values of innate immune response.

State variable	Susceptible person	Infected person	Exposed person
**U**_**H**__0_	5 × 10^8^	5 × 10^8^	5 × 10^8^
**U**_**E**__0_	0	3 × 10^3^	0
**U**_**I**__0_	0	1․5 × 10^3^	0
**U**_**R**__0_	0	0	0
**V**_0_	0	10^−3^	10^−3^
[**IFN**]_0_	0	0	0
**K**_0_	8 × 10^5^	8 × 10^5^	8 × 10^5^

## Data Availability

The data used are included within the paper and cited accordingly.
